The article "Seven Mathematical Models of Hemorrhagic Shock" was published in 2021. Journal: Comput Math Methods Med.

# Seven Mathematical Models of Hemorrhagic Shock

**DOI:** 10.1155/2021/6640638

**Published:** 2021-06-03

**Authors:** Luciano Curcio, Laura D'Orsi, Andrea De Gaetano

**Affiliations:** ^1^National Research Council of Italy, Institute for Biomedical Research and Innovation, Via Ugo La Malfa, 153, 90146 Palermo, Italy; ^2^National Research Council of Italy, Institute for Systems Analysis and Computer Science “A. Ruberti, ” BioMatLab (Biomathematics Laboratory), UCSC Largo A. Gemelli 8, 00168 Rome, Italy

## Abstract

Although mathematical modelling of pressure-flow dynamics in the cardiocirculatory system has a lengthy history, readily finding the appropriate model for the experimental situation at hand is often a challenge in and of itself. An ideal model would be relatively easy to use and reliable, besides being ethically acceptable. Furthermore, it would address the pathogenic features of the cardiovascular disease that one seeks to investigate. No universally valid model has been identified, even though a host of models have been developed. The object of this review is to describe several of the most relevant mathematical models of the cardiovascular system: the physiological features of circulatory dynamics are explained, and their mathematical formulations are compared. The focus is on the whole-body scale mathematical models that portray the subject's responses to hypovolemic shock. The models contained in this review differ from one another, both in the mathematical methodology adopted and in the physiological or pathological aspects described. Each model, in fact, mimics different aspects of cardiocirculatory physiology and pathophysiology to varying degrees: some of these models are geared to better understand the mechanisms of vascular hemodynamics, whereas others focus more on disease states so as to develop therapeutic standards of care or to test novel approaches. We will elucidate key issues involved in the modeling of cardiovascular system and its control by reviewing seven of these models developed to address these specific purposes.

## 1. Introduction

The quantitative understanding of the pathologic compensation to injuries is a key factor in improving the survival of trauma victims. In the process of devising enhancement for trauma care, and in particular for countering hemorrhagic shock, a thorough review of published contributions was a necessary first step. The present review reports the results of this investigation.

In the literature, there are a large number of mathematical models simulating human hemorrhage for different levels of blood loss from minimal to life-threatening or lethal. In general, understanding the time-dependent global hemodynamics is essential for predicting hemodynamic collapse and mortality after trauma and should be accounted for in mathematical models of the response to trauma.

In cases where trauma and hemorrhage lead to shock, relevant changes can occur on a relatively short time scale and typically involve acidosis/hypoxia, transcapillary refill, baroreflex control, etc.

The aim of our investigation was to select a certain number of representative mathematical models, models that succeed in reproducing the pathophysiologic response to hemorrhage, explicitly representing the most significant hemodynamic variables, those variables or indicators which medical doctors focus upon when interpreting the likely evolution of their patients and the effectiveness of the administrated therapies.

We believe that simulation technology combined with ever increasing data processing capacity may prove to be a decisive tool for understanding cardiocirculatory hemodynamics. By using computational models, experimental data can be interpreted more objectively. Model-directed experimentation serves not only to refine the models and identify their parameters but also to clarify the interpretation of other experimental results.

We can consider this process as a synergistic interplay between experimental and computational phases.

Since Grodins published his own global dynamic model in 1959, many mathematical models have followed [1]. The wide variety of such models differ in terms of their purpose and the methodology adopted.

Authors such as Frank [2], Guyton et al. [3–9], and Grodins et al. [1, 10] conducted experiments in their own laboratories, while others, like Beard et al. [11], Batzel et al. [12], and Zenker et al. [13], used reported results obtained from animal models. Still others, such as Siam et al. [14], relied mainly on theoretical models.

The choice of models reviewed here reflects our focus on the mathematical modeling of the response to hypovolemic shock. We selected whole-body scale models considering, as key hemodynamic variables, arterial and venous pressures, cardiac output, cardiac frequency, and stroke volume.

The structure of this paper is as follows: in the remaining part of the introduction, a very brief description of each of the considered models is given, in order to situate them in context, with respect to each other. In the overview section, a general classification of the existing models is offered, so that interested readers may rapidly focus their attention with regard to the chronological development and the functional and operational characteristics of the models. In Materials and Methods, a brief description of the procedure followed to identify and select the models is shown. In Results, each specific model is presented and discussed in detail: this section represents the main body of the current work. A short discussion comparing modeling approaches and some concluding remarks complete the paper.

As a universally recognized “standard” for the basic morphology of the arterial pressure pulse, the Windkessel model of the arterial tree [15] is described first. Furthermore, this model may also be considered a foundation for the other six models described [2].

Hemodynamic models of the circulatory system often employ “lumped-parameter” methods, assuming uniform distributions of pressure within vascular compartments. A zero-dimensional model (i.e., “lumped-parameter” model) may use an analogy with electrical circuits, where blood flow, viscosity, and pressure are analogous to current, resistance, and voltage, respectively.

According to this analogy, frictional losses are resistors, inertance of blood flow is represented as inductors (for large vessels), and vessel elasticity translates into capacitors. In electrical network analysis, Kirchhoff's current and voltage laws make it possible to determine voltage drops and current flows through every component of the circuit.

In its initial conceptualization as a 2-component Windkessel model, Otto Frank [2] devised a capacitor in parallel with a resistor. The former represented a reserve of “stressed” blood volume within large-vessel arteries, whereas the latter accounted for dissipative losses incurred as blood makes its way throughout the systemic circulatory tree. The appeal of “lumped-parameter” models is self-evident, given their mathematical versatility. In fact, they are both easily derivable and can be expressed as simple ordinary differential equations.

The second model that we illustrate, i.e., the Guyton, Coleman, and Granger model [3], is arguably the most popular and comprehensive circulatory-system model. Guyton's very extensive model has been in some sense the pioneer of the whole investigation into mathematical modelling of the circulation: it consists of many equations addressing most relevant aspects of total-body cardiocirculatory compensation by concentrating, in turn, on specific subsystems (renal, haemopoietic, thirst, cardiac pump, etc.) [3].

A salient feature of long-term blood pressure control is the dominant role of the kidney. The model describes the importance of renal control of blood volume in maintaining physiological blood pressures in response to perturbations, also quantifying response of the kidneys to such changes [3]. The importance of the SNS (sympathetic nervous system) in maintaining long-term blood pressure control is only marginally considered in the Guyton-Coleman-Granger model.

While extremely comprehensive, the model is very complicated, has not been validated on actual perturbation experiments, and is prone to adopt numerical shortcuts (thresholds, etc.).

In any case, the Guyton model remains the most widely studied cardiovascular model to date. Notwithstanding, it continues to fuel numerous debates [16] as to its validity in representing the human cardiovascular system [17, 18].

In 1959, Grodins [1] formulated a comprehensive mathematical model of the cardiovascular system. Two different circuits arranged in series compose this model: systemic circuit and pulmonary circuit. The left and right ventricles are instead represented by two pumps. The Grodins' model is a compartimental model in which arterial and venous storage volumes of the systemic and pulmonary circuits are two different compartments and, with mass balance equation, the relationships for blood inflow and outflow from the compartments are modeled [1].

With volumes equated to compartments, we have arterial and venous-storage compartments, i.e., systemic and pulmonary circuits, respectively.

The compartment equations involve mass balance relationships for blood inflow and outflow from the compartments. In this model, arterial blood pressure *P*_*as*_ and the baroreflex mechanism which acts to stabilize *P*_*as*_ during significant perturbations, such as hemorrhage, are taken into account by relationships between resistance and metabolic factors [1]. Embedded into the model for both the right and left ventricles, as measureable cardiovascular determinants, namely, *P*_*as*_, cardiac frequency *F*, systemic resistance *R*_*s*_, and cardiac output *Q* [1], their relationships can be expressed mathematically.

Batzel et al. [12] design their cardiovascular model based on Grodins' four-compartment model employing Starling's law of the heart and introducing the Bowditch effect [1]. The autonomic control system developed by the Authors acts on a single feedback loop and allows to evaluate the effect of hearth rate on stabilizing arterial pressure during a hemorrhage. In particular, this model proposes a baroreflex control system that allows the study of the characteristic changes in blood pressure and heart rate during and after acute blood loss of varying degrees of severity.

In order to evaluate oxygen delivery at physiological and at hemorrhagic conditions for different fluid resuscitation regimes, a hemodynamic model of the human adult cardiovascular system was developed by Siam et al. [14]. This model comprises a cardiovascular compartment and an interstitial compartment between which there is fluid exchange. It further represents the distribution of blood to different organ systems, the interaction among vascular beds, the blood pressure gradients, and blood flow and oxygen delivery throughout the cardiovascular system. The Authors' goal was to explore optimal fluid volumes and infusion rates so as to maximize tissue oxygen delivery rate of *D*_*O*_2__ [14]. As a secondary objective, they sought to define clinical markers (or endpoint) that could be monitored during fluid resuscitation so as to predict maximum *D*_*O*_2__ values [14].

Beard et al. [11], starting from the pressure-diuresis and pressure-natriuresis relationships considered by Guyton in his model [3], have developed a new model of long-term control of arterial blood pressure. In fact, Beard et al. assert that the “three laws of long-term arterial pressure regulation” of Guyton [19] constitute tautologies [20, 21]. Both baroreflex and renal mechanisms (i.e., the renin-angiotensin system) are factored into the model, thus their interactions with key effector organs, such as the vascular smooth muscle, heart, and kidney. The model is explicitly documented allowing for definition and reproducibility: all model equations are reported in the original publications and are validated based on experimental data. Parameter values are reported as well: all parameter values were estimated by comparing model simulations to measured data. This model is used to investigate the mechanisms that explain the chronic pressure natriuresis curves and to examine the mechanism by which the stimulation of the baroreflex reduces the arterial pressure. Hypotheses concerning the etiology of primary hypertension are also advanced [11].

Finally, we describe Zenker et al.'s model [13]. With respect to the currently available models, its outstanding feature is that it uses a simplified representation of the cardiovascular system and its control to simulate volume loss (e.g., hemorrhage). Notwithstanding its simplicity, it can portray the evolution over time of most clinically relevant variables, such as mean arterial pressure, heart rate, venous pressure, and cardiac output.

It consists of a continuous representation of the left heart, as a pump, the systemic circulation with the large arteries, treated as linear capacitors (as in the Windkessel model), with the arterial pressure controlled by a physiological feedback loop [2]. For purposes of simplification, the pulmonary circulation is excluded. His simplified 5-ODE model of the cardiovascular system is inclusive of baroreflex pressure control, with specific focus on the interactions between myocardial contractility, intravascular volume, and peripheral resistance.

Zenker et al.'s model is geared for simulation scenarios less concerned with intrabeat details, but instead mainly focused on continuous interbeat dynamics [13].

## 2. Overview

The present section offers a synthesis of the panorama of available cardiocirculatory models, organized systematically. This synthesis is mostly based on Kappel and Batzel [22] and Shi et al. [23] to which the readers refer for details.

In this section, we examine some key features concerning the modeling of the respiratory and cardiovascular control systems. Moreover, we summarily describe some of the significant models which have been generated to address these issues. The understanding of the underlying cardiovascular mechanisms and their control systems is sufficiently well understood to develop a number of mathematical models to try to explain their workings. However, cardiovascular control systems involve a complex set of interrelationships among such quantities as heart rate, blood pressure, cardiac output, and blood vessel resistance, such that the description of the control relationships is far from complete. We will consider several crucial areas of cardiovascular control and some milestones of the modeling approaches that have been used to elucidate the control processes. One approach to analyzing the cardiovascular and respiratory systems entails the application of optimality conditions, based on optimal control theory, into the design of these systems and the modeling process.

Mathematical models of the cardiovascular system may belong to several categories, such as the following [22]:

- Models of the mechanical cardiocirculatory system
- Models of control of the cardiocirculatory system
- Pulsatile versus nonpulsatile models
- Comprehensive versus restricted models
- Models classified according to dimensionality

The seminal investigation into the mechanics of the cardiovascular system by way of mathematical analysis dates back to 1899 with the work of Frank [2] and his followers, subsequently pursued by Aperia [24] and MacDonald [25]. Modeling of the mechanical system deals arterial and venous blood flow, the cardiac cycle, and other phenomena not involving active control processes [22].

Given the complexity of the entire cardiovascular system, many models have focused only on less comprehensive aspects, such as pressure-flow studies in arterial or venous compartments [25–45], left heart-artery studies [46–48], cardiac activity and circulation [49, 50], the baroreflex loop [51–54], local resistance autoregulation [55–57], resistance-pressure-flow relationships [58, 59], baroreflex control of heart rate variability [60, 61] and contractility [62, 63], or the influence of specific physiological states, such as sleep [64], or pathological conditions such as hemorrhage under different fluid resuscitation regimes [12, 14] or medical interventions [65]. The interrelatedness of the various mechanisms requires that models address the issue of meaningful simplification while bearing in mind the unitary nature of the system as a whole.

Arguably, the more a model includes the totality of constituent parts that make up the cardiovascular system, the more comprehensive it is defined. Conversely, local models are of narrower scope, focusing on a key feature or a discrete subset of these. By this criterion, a number of comprehensive cardiovascular system models have been developed. In turn, they are distinguished according to the nature of blood flow, as either pulsatile (involving effects determined by the cardiac cycle) or nonpulsatile, each incorporating one or more mechanisms of cardiovascular control [22].

Many comprehensive models of the cardiovascular system stem from Grodins' seminal four-compartment model presented in 1959 [1, 66]. It comprises both a systemic and a pulmonary circuit arranged in series, whereby the left and right ventricles are equated to pumps. Mirroring Grodins' respiratory model, the basic structure consists of compartments representing volumes, i.e., the arterial and venous blood storage volumes of the systemic and pulmonary circuits, respectively. The compartment equations define mass-balance relationships between inflow and outflow within and among compartments. Specifically, in Grodins' model, the control processes included interrelationships between peripheral resistance and metabolic factors affecting arterial blood pressure *P*_as_, along with baroreflex responses for stabilizing *P*_as_ perturbations, notably hemorrhage [22].

Notwithstanding its empirical underpinnings, it effectively provided the groundwork regarding the interrelationships among key cardiovascular variables, most notably: *P*_as_, heart rate *H*, systemic resistance *R*_*s*_, and cardiac output *Q* for both cardiac chambers [22].

Pulsatility is crucial to certain cardiovascular phenomena [67–73]. For example, pulsatile arterial blood flow results in a fairly steady distribution of blood to all tissues of the body, which could not occur otherwise. The role of pulsatility is also key to the baroreflex response to certain situations, as described by Ursino et al. [54]. However, since these pulsatile features are essentially superimposed on the underlying general flow, models using nonpulsatile flow more aptly lend themselves to other applications, e.g., pharmacokinetic studies. Similarly, whenever pulsatility has no decisive role, for example, when all the tissue compartments can be equated to a single compartment, the role of pulsatility con equally be overlooked. Indeed, Grodins' model is nonpulsatile as are subsequent models [74–77].

Another pulsatile model can be found in DeBoer et al. [78] who used difference equations. The latter describe how the features of one beat influence the characteristics of the next.

The model includes key cardiovascular parameters like (sympathetic) baroreflex control of heart rate and peripheral resistance and cardiac contractility. However, lesser contributors to blood pressure, such as those determined by the mechanics of respiration as well as Windkessel properties, are also incorporated [22].

The model was used to investigate short-term physiological variations in heart rate and blood pressure as well as the effects of specific pharmaceuticals. A noteworthy finding was the observation that the 10-second Meyer wave could be modeled in terms of a delay in the baroreflex loop. Studies of bifurcation, as described by Eyal and Akselrod [79], have also been based on this model.

Kappel and Peer instead adapted Grodins' model to study physiological transitions, such as from the resting state to physical exertion [80, 81]. Their model included a relationship between systemic resistance and local venous *O*_2_ concentration as described by Peskin [57], in turn based on the work of Huntsman et al. [82]. At steady state, heart rate *H* and contractility are related through the Bowditch effect, according to which cardiac contractility increases with increasing rates. Studies conducted by Kappel and Peer [80] demonstrated that any stability requires that contractility adapt to higher rates with a certain time lag.

Accordingly, a dynamical relationship between rate *H* and contractility was modeled via a second-order differential equation. The most significant aspect of Kappel and Peer's model was the introduction of optimal control as the crucial mechanism underlying arterial blood pressure control. In this approach, optimality refers to minimizing deviations in both blood pressure and energy requirements by penalizing extreme variations in heart rate, in turn acting as the ultimate controller. Through this “black box modeling” of the control systems for the baroreceptor loop, we can also determine the influence that the optimality criteria have on the entire yield of the system. Additionally, optimality criteria were applied to baroreflex function in Kappel and Peer [80, 81] as well as into a study of cardiovascular-respiratory control during exercise by Timischl [83].

Guyton and Coleman's comprehensive model was a milestone in cardiovascular modeling [84]. Since its primary concern revolved around blood pressure and the control mechanisms thereof, especially in hypertensive states, the model mainly focused on fluid regulation and thus renal function, ultimately [22].

Besides incorporating variable fluid volume and kidney function, the Guyton-Coleman model included the cardiac effects of hemodynamic load, autonomic reflexes (including baroreflex and chemoreflex function), and autoregulation of flow within tissue compartments [22].

Model simulations lent ample support for the preeminence of kidney function in the long-term control of arterial blood pressure. Recently, Beard et al. developed a model of long-term control of arterial pressure incorporating Guyton's concept of pressure-diuresis/natriuresis as physiological input-output relationships [11]. For other applications, such as short-term blood pressure control, fluid levels can be assumed constant; thus, kidney function needs not be taken into consideration (e.g., see [83]).

A number of models have limited their investigations into specific features of the baroreflex control loop or other control features. One such model by Kenner [85] represented the autoregulatory pressure and flow controls in the peripheral arteries as well as the baroreflex mechanism by first-order transfer functions. The latter allows for linear analysis of overall stability within the system.

Ursino et al.'s mathematical model [54] describes the effects of pulsatile flow on the hemodynamic properties and functioning of the cardiovascular system. Aside from the mass balance equations, the model also included representations of the cardiac pump, sympathetic control of heart rate, peripheral resistance, and pressure-volume relationships of systemic veins. Model simulations reproduced experimental findings, corroborating the role of pulsatility in carotid baroreflex control. Lafer studied the effects on cardiac contractions via sympathetic and parasympathetic nervous system interactions as well as the dependency of stroke volume on ventricular compliance [86].

The cardiac effects of time delay on baroreflex control have also been investigated by Cavalcanti and Belardinelli [87] and Ottesen [88]. Via simple mathematical models of short-term blood pressure control, these Authors analyzed stability properties subjected to one-second delay increases in the baroreceptor loop. In a recent mathematical model by Ursino [89], a range of important factors involved in the control of short-term arterial pressure were included. It consists in a six-compartment description of the vascular system with a model of the pulsating heart and two groups of baroreceptors, also accounting for SNS activity. Also included are the influence of arterial pressure (baroreflex), sympathetic activity, cardiac cycle, systemic peripheral resistance, and heart contractility. The model, whose results were consistent with experimental data, was used to simulate clinical scenarios involving baroreflex responses, among which are varying degrees of acute hemorrhage [22].

### 2.1. Combined Cardiovascular-Respiratory Models

The cardiovascular and respiratory systems are by no means independent of one another, but rather their functioning is largely the product of their interactions. The mechanisms for cardiovascular control interact with those for respiratory control causing delays due to transport time in the bloodstream between the lungs and the chemoreceptors (central and peripheral) that measure the levels of *P*_*a*_*CO*_2___ and *P*_*a*_*O*_2___, modified during the ventilation.

The rate and distribution of blood flow also influence the efficiency of gas exchange in the lungs and the function of tissue compartments. Vasomotor activity is related to respiratory center activity such that increases in its activity also tend to increase respiration. The recent model of the human respiratory control system by Ursino et al. [90, 91] incorporates several of these cardiorespiratory interactions, focusing on responses to hypoxic and hypercapnic stimuli. The model presented by Timischl [83] can be viewed as a combined and extended rendition of preexisting work by Kappel and Peer [80] and Khoo et al. [92]. This cardiocirculatory and respiratory model integrated some mechanisms in order to implement an optimal control.

Timischl et al. [64] further extended the model to include wake-to-sleep transitions and subsequently incorporated delays into the respiratory submodel [93]. Wabel and Leonhardt [94] also presented a model to simulate the cardiovascular and respiratory systems. Availing themselves of the MATLAB toolbox Simulink for their simulations, they redesigned the model devised by Coleman and coworkers. The heart, circulatory and respiratory systems, kidneys, and key nervous system control mechanisms, as well as humoral, i.e., endocrine, components, were all included [22].

### 2.2. Dimensionality

In function of the desired goals and accuracy of the study, models can be chosen according to varying dimensionalities in representation. In particular, the physiology of the cardiocirculatory apparatus can be studied through zero-dimensional (0D) and one-dimensional (1D) mathematical models. An underlying assumption of 0D models is the uniform distribution of the essential variables (i.e. pressure, flow and volume) regardless of the compartment (i.e., organ, vessel, or vessel segment) at any given time. In contrast, the higher dimensional models allow for variations of these parameters [23].

0D models are geared to evaluate the hemodynamic interactions of components of the cardiovascular system, in the whole cardiocirculatory system. Instead, 1D models can efficiently characterize pulse wave transmission in the arterial tree, at a fraction of the computational requirements of higher order computational modelling.

0D modeling is a theoretical useful frame that utilizes the concept of the hydraulic-electrical analogue. As hydraulic impedance takes into account the effects of the frictional loss, the elasticity of the vessel wall, and the blood inertia on the blood stream, the electrical impedance integrates the effects of resistance, capacitance, and inductance on the electrical circuits [23]. Blood flow is described via the continuity equation for mass conservation, whereas the flow of electrons in the circuit follows Kirchhoff's first and second circuit laws and Ohm's law.

Thus, conventional methods for analysis of electric circuits can be applied to investigate cardiovascular dynamics, where resistance *R*, inductance *L*, and capacitance *C* in the electric circuit describe the effects of friction, inertia, and vessel elasticity on blood flow, respectively. 0D cardiovascular modelling draws from Windkessel's original modeling of arterial flow, later employed to represent the heart, cardiac valves, and veins [23].

A host of 0D models has been spawned to describe specific characteristics of each circulatory subsystem. In terms of cardiovascular mechanics, a significant characteristic of 1D models consists in their capacity to depict wave transmission effects on the vasculature. Instead, two-dimensional (2D) models have a distinct role, relative to the vasculature, since they are well-adapted to representations of radial variations of velocity in axisymmetric tubes. In regions characterized by turbulence, the computing power of three-dimensional (3D) solutions is required to describe complex flow patterns. For detailed 3D cardiovascular flow modelling, see [49, 95–99]. “Lumped-parameter” models can be categorized by complexity, from the minimally complex (e.g., Windkessel models) to the extremely complex that may even include autonomic and endocrine feedback loops (e.g., the 1972 Guyton model) [3]. One classification divides the models into subgroups, namely, single- and multicompartment models.

In single-compartment models, the aggregate vasculature system, or its subsystems, can be reduced to one or more resistance-compliance-inductance (RLC) combinations (according to the anatomical distribution considered). The single-compartment prototype was the seminal two-element Windkessel model, originally designed by Hales in 1733, then mathematically formalized in 1899 by Otto Frank [100]. The Windkessel model has two components in parallel, a capacitor *C* emulating the storage function of large elastic arteries and a resistor *R* that equates to peripheral resistance vessels [23].

Albeit simple, RC combination models still have practical applications in the clinical setting. For instance, knowing peripheral resistance and the aortic pressure pulse waveform, overall arterial compliance can be calculated [100, 101]. In addition, it is often used in cardiovascular modeling to represent afterload, notwithstanding the limit of having a single time constant. To simulate added arterial features, Landes [102] further elaborated the Windkessel configuration by introducing the resistance *R*_*c*_, in series with the RC Windkessel model. Westerhof and coworkers extensively focused on this model, alternatively referred to as the Westkessel model, or RCR model [102]. The added resistance *R*_*c*_ stands for the typical impedance of the arterial network [103], representing a significant improvement in high frequency performance [102]. The sum of the resistances *R*_*c*_ + *R* equates to the total systemic vascular resistance of the previous (Windkessel) RC model, while the capacitance *C* accounts for the mechanical elasticity of the arterial vascular bed [102].

However, the RCR model has demonstrated a number of shortcomings, in *in vivo* studies. In particular, the latter include underestimations of peak aortic flow and mean arterial pressure, of significant degree for the former, yet marginal for the latter. In addition, aortic pressure and flow waveforms result entirely unrealistic. Nevertheless, the RCR model is still widely employed in cardiovascular modelling, with reference to afterload, to evaluate cardiac functioning in a host of physiological or pathological settings [104].

Concurrently to the Westkessel RCR model, Burattini and Natalucci developed their own [105]. To describe the arterial features, the latter adopted an alternative configuration of the three-element RCR model. In it, a small resistance *R*_*c*_ was used in series, not with the RC combination, but rather with the capacitor *C*. Conceptually, this coupling of the small resistance *R*_*c*_ to the capacitor *C* should account for arterial viscoelasticity [23].

With the introduction of the aforementioned inertial term *L*, the vessel impedance calculation is more precise in the midfrequency spectrum. In detail, by integrating the inertia of the blood flow via a RLCR1 model, Landes [102] succeeded in enriching the RCR model. In particular, by incorporating the inertial effect of blood flow via a RLCR1 model configuration, Landes [102] succeeded in enriching the RCR arterial model. Likewise, Westerhof et al. also incorporated the inertial effect of blood flow into the RCR model, obtaining however an altogether diverse RLCR2 four-element arterial model [106, 107].

A number of independent comparative *in vivo* studies, specifically designed to test modeling accuracy of the RC, RCR, RLRC1, and RLRC2 models, have demonstrated the RLRC1 model to perform best [108]. For most applications, RC, RCR, and RLRC1 models adequately address overall hemodynamics. In fact, in circulatory beds such as the aorta and major vessel branches, venous pressure and pressure pulsation are negligible. However, in the coronary and pulmonary circulatory beds, the venous contribution must also be considered [109].

In single-compartment models, the entire systemic vasculature represents a single block, thus eliminating the need to compute pressures and flow rates of individual branches. On the contrary, in multicompartment models [110–115], each segment or compartment has its own resistance *R*, compliance *C*, and inductance *L*, depending on the local characteristics, which are then compiled into a unified model of the whole network system. For each study, the models can be tailored to suit the specific region(s) of interest and required accuracy. For each study, the models can be tailored to suit the specific region(s) of interest and required accuracy [23].

The building blocks for the development of vessel network models, in multiple-compartment models, consist in suitable RLC models for each vessel segment [110, 116].

In particular, Formaggia and Veneziani [117] and Milisic and Quarteroni [118] provided formal derivations of four compartment model configurations capable of describing individual vessel segments from which several multicompartment models have been developed, spanning from single branch models to those of greater complexity. Generally, researchers partition the systemic vasculature into segments of every caliber [54, 69, 119] and then connect the segments into a loop.

In order to investigate blood-flow distribution and pressure/flow curves in individual simulated vessel branches, other Authors have designed multibranch, multicompartment models [110, 116, 120–123]. For full-body models for the systemic arterial network, see [123–125].

Increasingly sophisticated and advanced configurations of 0D models have had widespread applications as reliable tools in the study of cardiovascular physiology. Although 1D models have been traditionally confined to the study of arterial hemodynamics, more recent applications in the clinical diagnosis of cardiovascular pathology (e.g., arterial hypertension and atherosclerosis) have been successful [23].

Since overly simple models generally have unsatisfactory accuracy, the researcher must often accept a trade-off between level of model sophistication and its reliability, according to the investigator's specific needs. Since 0D cardiovascular models, especially those of higher complexity, are essentially intended for research, it comes as no surprise that few integrated 0D models have had clinical applications [23].

## 3. Materials and Methods

After a comprehensive literature search on cardiovascular modeling in PubMed, Google Scholar, Ovid, ScienceDirect, and Cochrane Library search engines, we selected seven models that we deemed representative of the category of circulatory models able to simulate hemodynamic responses to hypovolemic shock, at the whole-body scale.

The global hemodynamics models typically consist in a closed-loop hydraulic circuit. The various components of the body are represented as lumped, i.e., zero-dimensional and descriptions, with bleeding as an option.

As regards the constitutive equations of the models, these will be concisely described. Moreover, authorship of diagrams and graphs herein included or cited are duly acknowledged in the references to the original papers. For each work, the mathematical notations, along with any tables, are reported as used by the Authors. Developing a uniform notation for all the models described in the present review would have proved challenging and not always possible.

## 4. Results

This section is dedicated to the description of the chosen models.

### 4.1. Windkessel

Mathematical modeling and parameter estimation may help to understand the cardiovascular system but is hampered due to the dynamic interactions within the vascular tree. A well-known approach to operationalizing cardiovascular modeling is via the Windkessel models (WM). The 2-element Windkessel model (2WM) considered in this discussion dates back to 1899. It is the first lumped-parameter arterial model designed by the German physiologist Otto Frank in 1899 [2].

According to this model, the human systemic arterial tree works as an elastic reservoir which, through the aortic valve, receives blood from the left ventricle, in a pulsatile manner, and supplies blood to the arterioles and capillaries, viewed collectively as being equivalent to vascular resistance. Downstream to microvascular bed (capillaries), we have the systemic venous circulation, which is attributed a value of zero pressure. In its most simplified form, we may consider the following one-tank model (Figure 1):

In this model formulation, *Q*_ao_ is the instantaneous aortic flow; *p* is the pressure in the tank, which is constant in every point and representative of aortic pressure; *V* is the volume of the reservoir, representative of the volume of blood contained in the arteries; *C* is the compliance of the tank ( = *dV*/*dP*), representative of the total arterial compliance; *p*_*v*_ is the venous pressure; and *R* is the peripheral resistance, defined as the ratio between the drop of arterio-venous pressure (*P* − *P*_*v*_) and the flow rate flowing through the arterioles and capillaries, assuming that the volume *V* is a linear function of pressure *P* (i.e., *V* = Vo + *C* · *P*), where Vo is a constant equal to the volume of the tank at zero pressure. Then, it is possible to write the overall volume for the tank as follows:

(1) $$\begin{array}{c} C\frac{dP}{dt}=Q_{\text{ao}}-\frac{P-P_{v}}{R},\;\text{with }P_{v}=0. \end{array}$$

The corresponding electrical analog may be considered as follows (Figure 2) with the corresponding differential expressed by the equation:

(2) $$\begin{array}{c} C_{\text{ar}}\frac{dP_{\text{ao}}}{dt}=Q_{\text{ao}}-\frac{P_{\text{ao}}}{R_{\text{per}}}. \end{array}$$

In essence, it consists of two lumped parameters, i.e., resistance *R* and compliance (alternatively labeled capacitance) *C* which are both ascribed to blood vessels. The effectiveness of the use of WM is based on the direct correspondence between these electrical components and their intrinsic physiological value. In fact, according to the law of the Hagen-Poiseuille (nonideal fluid dynamics), the resistance is strictly dependent on the radius of the blood vessel and the compliance represents elasticity. Large vessels represent compliances, whereas smaller vessels are equated to resistances.

Resistance vessels in the arterial tree are mainly represented by small arteries and arterioles, whereas *C* is mainly determined by the elastic properties of large vessels, predominantly the aorta. The 2WM thus provided insight into the contribution of the different arterial properties to the workload of the heart. The 2WM also provided the basis for different methods of estimating *C*, such as the decay time method [2], the area method [126, 127], and the pulse pressure method [128]. However, the 2-element model is of limited value in mimicking systemic input impedance (*Z*_in_) [107]. Also, when aortic flow is used as an input, this model produces unreliable wave shapes of aortic pressure and flow [107, 128]. This is mainly due to the poor representativeness of the aortic *Z*_in_ at frequencies in the medium to high range. To overcome this known weakness of the 2WM, Westerhof et al. [129], on the basis of new information about *Z*_in_, introduced the 3WM.

In the latter model, an additional resistance *Z*_*c*_ is added. It stands for the characteristic impedance of the proximal part of the arterial bed (aorta) and is subsequently applied to the same electrical circuit as the classic 2-element model. Borrowing from electronics, the concepts of characteristic impedance of the transmission medium and of *Z*_*c*_ propagation velocity of a wave, and taking into account the reflection properties of the waves, we can state that physiologically *Z*_*c*_ integrates the capacitive and inertial effects of the proximal ascending aorta. It is derived from transmission-line models and allows to adjust for the above-mentioned weakness. *Z*_*c*_ is connected in series with the 2-element windkessel circuit. The corresponding electrical analog is considered in Figure 3, and the relative equations are as follows:

(3) $$\begin{array}{c} C_{\text{ar}}\frac{dP_{\text{ac}}}{dt}=Q_{\text{ao}}-\frac{P_{\text{ac}}}{R_{\text{per}}},\\ P_{\text{ao}}=P_{\text{ac}}+Z_{c}\cdot Q_{\text{ao}}. \end{array}$$

The introduction of *Z*_*c*_ considerably improves the model at medium to high frequencies. As a consequence, the 3WM model produces more realistic pressure and flow wave shapes and a better fit with experimental data [107, 129, 130]. The 3WM is thus based on hemodynamic principles and has become the conventional lumped-parameter model of systemic circulation. Nevertheless, this model still presents some limitations when compared to experimental data [129]. In particular, *C* tends to be overestimated and *Z*_*c*_ underestimated.

In order to reduce the above errors in the low frequency range, owing to the characteristic impedance, the addition of a fourth element in the Windkessel circuit has been proposed [131], although originally introduced by Burattini and Gnudi [132]. The 4-element Windkessel model (4WM) thus expands the 3-element WM with an inertance *L*. The latter was placed in parallel with the characteristic impedance to form the 4WM thus consisting of two dynamic elements. Consequently, we need two states to describe its dynamics. The state vector consists of states *F*_*l*_(*t*) and *P*_*ac*_(*t*) with *F*_*l*_(*t*) denoting flow through the total arterial inertance. Again, assuming *Q*_*ao*_(*t*) as an input, the state equations are derived from the 4WM in the figure below.

The relative equations are as follows:

(4) $$\begin{array}{c} C_{\text{ar}}\frac{dP_{\text{ac}}}{dt}=Q_{\text{ao}}-\frac{P_{\text{ac}}}{R_{\text{per}}},\\ L\frac{dF_{l}}{dt}=Z_{c}\left(Q_{\text{ao}}-F_{l}\right),\\ P_{\text{ao}}=P_{\text{ac}}+Z_{c}\left(Q_{\text{ao}}-F_{l}\right). \end{array}$$

This fourth element (Figure 4) is an inertance equal to the sum of all inertances in the arterial segments, i.e., total arterial inertance [131].

The impact of total arterial inertance is mainly limited to the mean term. Similarly, it affects input impedance only for very low frequencies. This is important due to the fact that this is the very range where the 3-element WM lacks precision.

Other researchers have instead introduced an inertance in series with the characteristic impedance [108, 132–135]. Whereas high frequencies would affect arterial-input impedance with this series inertance, such effects do not occur at low frequencies. Although the inertance theoretically implies an increase in the impedance modulus in the high-frequency range, the inertance adopted minimizes those effects at low frequency. Of note, Segers et al. [136–138] and Burattini and Di Salvia [133] also adopted the 4-element WM. In practice, inertance results are quite difficult to estimate which is the rationale for preferring the 3-element WM. This 4-element model nevertheless offers undeniable advantages: it accounts for the inertia of the whole arterial system; it permits *Z*_*c*_ to come into play at the full spectrum (low, medium, and high) of frequencies.

### 4.2. Guyton

The pioneering work of Guyton et al. [3] (henceforth referred to as G72) which perform an analysis of the overall regulation of the cardiovascular system constitutes the first physiological model characterized by a functional integration (or horizontal integration) [139]. The Authors represented their mathematical model through a series of components functionally combined to simulate the key subsystems underlying the physiology of cardiovascular regulation. This model enables a multiorgan analysis of the regulation of the overall cardiovascular system capable of exploring events over time intervals, ranging from seconds to weeks or even months [139].

Guyton initially strived for extreme simplicity in devising his model of the cardiovascular system. He focused on the role of blood volume and vascular capacity. Thereby, he modeled a closed hydraulic loop that, at the same time, was able to account for short-term regulation of cardiac output. Subsequently, Guyton directed his efforts towards long-term regulation of arterial pressure. For the latter, two slow-acting mechanisms were deemed crucial: (1) the capacity to determine wide fluctuations in urinary output at relatively constant blood pressure (corresponding to the renal function curve, in Guytonian terms) and (2) long-term vascular autoregulation (i.e., changes in the extent of vascularization, constriction, or dilation of existing vessels) so as to adapt blood flow to meet oxygen demand in tissues [140]. At this second-stage, the model better explained the transient dynamics and steady state of renal hypertension. The third version of Guyton's model was further enriched by endocrine and neural facets, whose parameters have an established bearing on the renal function curve [140].

The G72 model consists of 18 modules (comprising over 350 elementary components), including approximately 160 variables, more than 40 of which constitute variables of state (cf. diagram in Guyton et al. [3, 141]). The model contains a total of approximately 500 values (i.e., model variables, parameters, and constants) [139].

Conceptually, Guyton constructed his original model around a “central” hub (called circulatory dynamics module) interacting with 17 spokes (peripheral modules) each corresponding to a separate physiological function [139].

Upon examination of the original code and published diagram, one may notice that, besides its interconnected module structure, the model allows for a wide range of time scales in the individual modules, spanning from intervals as short as 5 × 10^−4^ min (characteristic of autonomic control) to as long as 10^4^ min (that is, timeframes typical of chronic degeneration or remodeling, e.g., cardiac hypertrophy) [139]. Specifically, long-term regulatory effects on cardiovascular activity (the foremost of which represented by the renin-angiotensin-aldosterone axis) adopt time constants in the order of hours or days, whereas short-term regulation (most notably, baroreceptor reflexes) is more aptly measured in seconds.

The simulations obtained via the G72 model were used to perform simultaneous analyses of the main effects resulting from several types of stresses on the cardiovascular system [139]. Moreover, these simulations were even used to predict patterns of physiological behaviors that would have taken years to observe experimentally *in vivo* [139]. It also served to identify parts of the system where knowledge was still lacking, thus helping in the design of further research. Overall, however, the model has a merely descriptive value of the workings of cardiovascular system regulation. The foremost limits of the model consist in the impossibility to take into account most of the pathologies of interest.

Building on the foundation of the Guyton model, various Authors, such as Ikeda et al., designed more sophisticated versions. Ikeda et al. [142], however, included acid-base regulation parameters and variables (i.e., inputs/outputs), contemplating a host of solutes and metabolites. In addition, the respiratory subsystem, which is functionally interrelated with the subsystem regulating acid-base balance, was in turn based on a model provided by Grodins et al. [66, 143]. The three generations, i.e., evolutionary stages, of Guyton's model were described by Sagawa [140].

#### 4.2.1. First Generation of Guyton's Model of the Circulatory System

Guyton envisioned the entire hydraulic loop of circulation as opening at the vena cava-right heart junction, analyzing it at two ports, i.e., the atrium and vena cava [144] (cf. Fig. 1 in Sagawa [140], p. 260). In this way, both ports were forced via a single flow, which was the only way to maintain the total blood volume constant in the open loop. Thus, two curves could be derived from this open-loop analysis: one curve derived from the atrial port, describing the relationship between cardiac output and right atrial pressure (the Starling curve for cardiac output), and another curve from the vena cava port, pertaining to the relationship between venous return and right atrial pressure (i.e., the venous return curve). In a closed-loop system, the steady-state cardiac output and venous return equal each other [140]. Consequently, the intersection between the two curves was used to find the equilibrium point for cardiac output and venous return as well as for right atrial pressure in the closed-loop system. The venous return curve was based on a simplified model of the systemic vascular bed consisting only of resistances and capacitances for the arterial and venous compartments, respectively [140]. In this system, one of the most important parameters is represented by blood volume.

Via the total vascular capacity parameter, the blood volume determines the static filling pressure which can be measured in the absence of flow within the system. It is represented by the ordinate intercept of the venous return curve (cf. Figs. 1–2 in Sagawa [140], p. 260). The relationship allowed a graphic representation of how variations in blood volume, vascular resistance, and capacity in arterial or venous compartments, along with several other physiological and pathological perturbations, affect the equilibrium point, i.e., cardiac output and mean right atrial pressure [145].

#### 4.2.2. Second Generation of Guyton's Model of the Circulatory System

It is noteworthy that systemic arterial pressure was absent in the foregoing equilibrium diagram (First-Generation Model) [140]. Initially, Guyton focused mainly on cardiac output and its regulation [146]. Yet, arterial pressure is nevertheless the most frequently measured variable in experimental and clinical settings. Arterial hypertension directly or indirectly underlies significant cardiovascular morbidity and mortality in developed countries. Mean arterial pressure is the product of cardiac output and total systemic vascular resistance. The typical clinical picture of chronic hypertension is accompanied by significantly increased total peripheral resistance notwithstanding the apparently normal cardiac output [140, 147].

Based on the above considerations, the second stage of Guyton and his coworker's analysis [148] addressed this prominent health issue. They identified sequences of cardiovascular and renal events whose physiological interactions could give rise to patterns of chronic hypertension within a week or two. By tweaking parameters of renal function and urine output, desired increases in blood volume and thus cardiac output could be achieved within several days [140]. The increased cardiac output elicited rises in arterial pressure, which in turn increased urine production so as to match exogenous fluid intake [140]. Ultimately, a new point of equilibrium is reached at a higher arterial blood pressure and cardiac output, with an increase in total blood volume (cf. Fig. 4 in Sagawa [140], p. 261).

Two noteworthy features are, on the hand, the slope of the curve, whose steepness determines significant decreases in urinary output even with minimal pressure reductions at the renal artery, and on the other hand, the fact that marked increases in blood and interstitial fluid volumes can eventually result from reductions in urine output that are relatively minute, with respect to overall fluid intake. This time-dependent process is represented by the integrator illustrated in the diagram [140]. The increases in blood volume in turn manifest as increases in cardiac output and thus arterial pressures. Over a period of days, these events constitute an integrating-type negative feedback loop that controls urinary output with respect to water intake, so as to maintain a balance between water intake and urine output [140].

The system (cf. Fig. 5 in Sagawa [140], p. 261) shows that the renal manipulations produce rightward shifts in the renal function curve, whereas the equilibrium state (cf. Fig. 4 in Sagawa [140], p. 261) exhibits that a considerable increase in blood volume and cardiac output must be produced before arterial pressure rises sufficiently to balance urinary output with water intake by this rightward shift of the renal function curve alone [140].

Consequently, Guyton incorporated into his model a crucial hypothesis, which had no relationship with the renin-angiotensin system. According to the underlying hypothesis regarding the microvasculature, blood flow in excess of local tissue demands for oxygen automatically and proportionally increases resistance, with inverse effects on blood flow (i.e., oxygen supply). Although the onset of the postulated autoregulatory control of resistance vessels takes seconds or minutes, it may last for hours, if not days [140]. It involves both acute and chronic changes in vascular diameter but also in vascularization, via variations in the density of microvessels in tissues (cf. Fig. 6 in Sagawa [140], p. 262); it illustrates how the autoregulation is. The long-term autoregulatory (incorporated into Guyton's model) increase in total peripheral resistance also persists as a significant hypothesis in Guyton's third-generation model [140].

#### 4.2.3. Third Generation of Guyton's Model of the Circulatory System

In the latest generation of Guyton's model [3, 141] of circulation, the pathogenesis of renal hypertension maintains its pivotal role. Meanwhile, many studies of physiology continued to add to the knowledge regarding the workings of the renin-angiotensin-aldosterone system, elements of which were embedded into the third generation model [149]. Among the latter, we recall the role of autonomic nervous control of salt and water balance, including the thirst mechanism and the control of ADH release via vascular mechanoreceptors as well as via central osmoreceptors. In addition, renal sympathetic vasomotor reflexes were also taken into account [140].

That being said, critics of Guyton's model note its shortcomings as regards its limited contribution to our understanding of the pathophysiology of circulation [140]. Certain limitations can be defined *nonspecific* to the Guytonian model, although further amplified by the sheer bulk of the model itself. In fact, however detailed, it remains an extreme over simplification of the reality of the cardiovascular system.

The details of the dynamics at the cellular level would have to be incorporated into the model in order to account for the effects of thermoregulation, physical exertion in heat or cold, shock, the effect of gravity on cardiac output, and arterial pressure, just to name a few. These complex situations cannot predict by the model. Similarly, the effects on blood volume distribution of common perturbations such as epinephrine infusion allow rough approximations, at best [150, 151]. To its favor, however, the strength of the Guytonian model consists in its potential for simulating long-term phenomena as regards control mechanisms of arterial pressure and the dynamics of blood and interstitial fluid volume, via a formal model. As with any predictions, they are as valid as the underlying assumptions regarding the structures and parameters. However, the probability of obtaining valid conclusions is inversely proportional to the number of the incorporated assumptions. Therefore, for large-scale models such as Guyton's, it is crucial to avail oneself of as many experimentally established findings as possible concerning the interrelationships and the parametric shifts of each component of its subsystems. Guyton was quite cognizant of these inherent limitations, as exemplified by the following quote [3]:

*An important factor that allows a systems analysis such as this to predict actual function with good accuracy is the extreme stability of the actual circulatory control system. Because of this stability, the function of any single block, or of any single control mechanism, can be in error as much as*  ±50  *percent (sometimes even more than this) without significantly affecting the overall output of the system. . . ., If it were not for the extreme stability of the overall circulatory control system we would have to know far more basic physiology to make such a systems analysis as this work* [3].

One interpretation of the above statement highlights that the overall stability of arterial pressure and cardiac output *in vivo*, in the face of significant perturbations to individual components of the circulatory system, is paralleled in their model, despite wide fluctuations in parameter variations. In the ultimate analysis, it likely characterizes the essential features of the cardiovascular system to a sufficient degree of accuracy [140]. Accordingly, when the model registers marked departures from equilibrium, whether in pressure or flow, serious concern appears warranted. However, the inherent difficulties in accurately tracking the internal workings of a complex system through a limited set of variables are all too obvious [140]. Despite these challenges, Guyton's group delved into this real-world system and experimentally corroborated the structural and parametric values of their formal models with some degree of success [140]. Specifically, the most important, although least supported experimentally, hypothesis in Guyton's model is the long-term autoregulatory increase in total systemic resistance, whereas its counterpart, i.e., autoregulatory decreases in vascular resistance following sudden drops in tissue perfusion, is well documented in both animal and human experiments (see Coleman, et al. [152]).

A more advanced version of G72, originally created in 1992, was eventually stabilized. Despite never being published as such, it subsequently became the flagship version for Guyton's group, surviving in Fortran and C within his group, but was also adopted by other teams, even with a rather sophisticated command-line user interface in MS-DOS (MODSIM [153]).

The G72 model has the advantage of having a formal description as well as having adequate experimental data regarding its various components. However, the Guyton models, together with their subsequent versions [154], do not account for pulsatile cardiac function.

This poses major limitations, for instance, when studying heart failure (HF) inasmuch as [155]:

1. There is an inability to adequately represent the systolic and diastolic characteristics of HF and biventricular desynchronization
2. The maximum arterial pressure derivative, as well as other useful clinical variables, eludes being simulated
3. More realistic representations of short-term regulatory loops (such as the baroreceptor reflexes) inexorably rely on such pulsatile variables

### 4.3. Grodins

Most comprehensive models for the cardiovascular system stem from Grodins' four-compartment model, presented in 1959, as extensions or modifications thereof [1, 66]. This model is a *resistive-capacitive* model composed of three basic blocks: two pumps representing left and right hearts and a block representing the systemic and pulmonary circuits as depicted in Figure 5.

Analogous to Grodins' respiratory model, the basic model structure consists of compartments representing volumes. In particular, the volumes are the arterial and venous blood storage volumes of the systemic and pulmonary circuits. Mass balance relations for blood flow inputs and outputs of the compartments underlie the compartment equations [1].

In the model, there are also some control processes obtained by implementing a baroreflex mechanism by which it is possible to stabilize the arterial pressure *P*_*as*_ during possible traumatic events (e.g., hemorrhage). Furthermore, there are relationships between systemic resistances and metabolic factors that allow the analysis and understanding of the interrelations of some of the most significant hemodynamic variables: arterial pressure *P*_*as*_, heart rate *H*, systemic resistance *R*_*s*_, and cardiac output *Q* for both hearts [1].

Here, we illustrate the fundamental equations of the model considering the simplification proposed from Noordergraaf in his passage [156].

The purpose of Grodins is to simulate the steady-state conditions of the cardiovascular system considering the Frank-Starling law as the basis of the description of the behavior of the heart. Therefore, the volume work performed by the heart is [1]:

(5) $$\begin{array}{c} w_{s}=Sv_{d}. \end{array}$$

*S* is the proportionality constant that represents the “strength” of the ventricle, and *v*_*d*_ is the diastolic volume. *w*_*s*_ can also be expressed as the product of stroke volume *v*_*s*_ and mean arterial pressure *P*_*A*_ [1]:

(6) $$\begin{array}{c} w_{s}=v_{s}P_{A}. \end{array}$$

Rest volume *v*_*r*_ is defined as [1]:

(7) $$\begin{array}{c} v_{r}=v_{d}-v_{s}. \end{array}$$

Ignoring the atrial contributions and posing that the ventricular relaxation occurs immediately at the end of the systole, that the filling of the relaxed ventricle is a linear process driven by a constant venous pressure and hindered by internal viscoelastic frictions, and that the unstressed volume of the relaxed ventricle is zero, Grodins' ventricular filling law is obtained [1]:

(8) $$\begin{array}{c} RC{\dot{v}}_{d}+v_{d}=CP_{V}, \end{array}$$

describing the relationship between diastolic volume at time *t*(*v*_*d*_), venous filling pressure (*P*_*V*_), compliance of the relaxed ventricle (*C*), and total viscous resistance (*R*).

Assuming *R* and *C* linear and time-invariant, since at *t* = 0, *v*_*d*_=*v*_*r*_, the solution of the previous differential equation is [1]:

(9) $$\begin{array}{c} V_{d}=CP_{V}+\left(V_{r}-CP_{V}\right)e^{-t/RC}. \end{array}$$

In steady-state conditions, for an isolated ventricle, assuming a constant systole duration of 0.2 s, the duration of filling *t* is assumed to be related to dependent on heart rate *n* (cycles per second) and it is defined as [1]:

(10) $$\begin{array}{c} t=\frac{1}{n}-0.2. \end{array}$$

The cardiac output *Q* is given by [1]:

(11) $$\begin{array}{c} Q=nv_{s}. \end{array}$$

The set of equations (5)–(11), hold for both hearts, with equation (10) in common, represent eleven independent equations. Instead of considering the complete vascular tree, we have the peripheral flow given by [1]:

(12) $$\begin{array}{c} Q_{\text{per}}=\frac{P_{A}-P_{V}}{R_{\text{per}}}, \end{array}$$

where *R*_per_ stands for peripheral resistance. The pressure-volume relationship on the arterial side is [1]:

(13) $$\begin{array}{c} P_{A}=\frac{1}{C_{A}}V_{A}, \end{array}$$

and on the venous side [1]:

(14) $$\begin{array}{c} P_{V}=\frac{1}{C_{V}}V_{V}. \end{array}$$

Defining [1]:

(15) $$\begin{array}{c} B=V_{A}+V_{V} \end{array}$$

and taking into account that these 4 equations are valid both for the systemic and for the pulmonary circuit, another 8 equations must be added and so the number of independent equations rises to 19.

Considering the steady-state restrictions under which the system will operate (i.e., the flows outgoing from the right and left heart must be equal to each other and at the same time equal to the flows in the systemic and pulmonary circuit) [1]:

(16) $$\begin{array}{c} Q_{L}=Q_{R}\equiv Q,\\ Q_{L}=F_{S},\\ Q_{R}=F_{P}, \end{array}$$

moreover, it must be considered that the total amount of circulating blood is equal to the sum of the blood present in the systemic and pulmonary tree [1]:

(17) $$\begin{array}{c} B_{T}=B_{S}+B_{P}. \end{array}$$

In this way, 4 more equations are added to the previous 19, bringing the total number to 23.

The given set of equations describes the Grodins model, a mathematical model by which it is possible to describe the cardiovascular system. Grodins is one of the first scholars to have experimented with the use of computers in the analysis of physiological phenomena affecting the human body, in particular the cardiorespiratory system.

We want to recall that Grodins' pioneering work began in the 1950s when he first suggested the use of control theory to explain the respiratory system and its regulatory mechanisms. In 1954, Grodins presented his seminal work [157] in which the respiratory system is represented as a closed-loop feedback system.

### 4.4. Siam

For the purpose of simulating and evaluating arterial oxygen delivery at normal and at hemorrhagic conditions under different fluid resuscitation regimes, a hemodynamic model of the human adult cardiovascular system was developed by Siam and his colleagues [14, 158]. By way of the model, hematocrit and mean arterial pressure can be used to optimize infusion rates and volumes for effective resuscitation maneuvers. The calculations thus identify the optimal fluid replacement regimen required to assure maximal oxygen delivery rates at the given conditions of controlled bleeding [14].

Cell necrosis ultimately leading to multiorgan failure occurs only in the end stages of severe hemorrhagic hypovolemia [159–161]. These, however, result from a cascade of systemic events that alter hemodynamic parameters and blood composition, ultimately impairing oxygen delivery to vital organs [14]. Another matter of debate concerns the optimal volumes and rates of fluid replacement. Various animal models have been developed to address the effects of various fluid volumes and rates on mortality and rebleeding endpoints [162–165]; nevertheless, the optimal fluid resuscitation protocol remains elusive [14].

The Authors designed a mathematical-model study to explore optimal fluid volumes and infusion rates so as to maximize tissue oxygen delivery *D*_*O*_2__ rate [14]. Another objective was to define clinical markers (or endpoints) that could be monitored during fluid resuscitation so as to predict maximum *D*_*O*_2__ values [14]. The physiological underpinnings of such an optimal point (i.e., of maximal *D*_*O*_2__ rate) are the inverse effects of fluid administration on cardiac output (CO) and hematocrit (HCT), which are the two major determinants of oxygen delivery [14]. In the context of fluid replacement therapy, the temporal dynamics of tissue oxygen delivery rate were elucidated. Such studies served to establish effective fluid-replacement protocols of infusion rates and volumes, i.e., capable of assuring continuous and maximal oxygen delivery. Furthermore, the impact of fluid type (i.e., crystalloids or colloids) on the hemodynamic responses and oxygen delivery to tissues was also studied [14].

Their hypothesis revolved around the notion of the existence of an optimal value of oxygen delivery, where fluid administration could be interrupted. The latter point could be established in the field using HCT and mean arterial pressure (MAP) values as the two main determinants of oxygen delivery [14].

#### 4.4.1. Description of the Model

The model structure (cf. Fig. 1 in Siam et al. [14], p. 84) is based on prior model versions [166]. We can see that the system comprises separate compartments: a cardiovascular compartment and an interstitial compartment, between which there is fluid exchange. It is a structural representation of the distribution of blood to different organ systems, the interaction among vascular beds, the blood pressure gradients, and blood flow and oxygen delivery throughout the cardiovascular system [14].

The cardiovascular model aimed to reproduce hemodynamic responses under conditions of hemorrhage and fluid resuscitation. The system model is subdivided into heart, a systemic circulation, a pulmonary circulation, and an interstitial compartment. The intravenous fluid load, flow, CO, and capillary pressure levels (i.e., rates of fluid exchanges between the intravascular and interstitial compartments) could be readily simulated [14]. The structural and mathematical aspects of the model: pressure, flow, and volume of individual chambers throughout the cardiac cycle are illustrated in Table 1 (cf. Tab. A1 in Siam et al. [14], p. 92). The model consists of multiple elements. Specifically, the aorta is subdivided into nine anatomical segments representing the aortic root, the arch, four thoracic aorta segments, and three abdominal aortic segments, respectively [14]. Each aortic segment in turn consists of a three-element circuit mimicking viscosity, fluid inertia, and vessel compliance, respectively [14]. Finally, the aorta gives rise to seven arterial branches that correspond to the relevant anatomical vasculature. Each arterial segment terminates with a capillary bed-equivalent resistor connecting the systemic arterial circulation to the corresponding venous circulation [14].

Each systemic artery/systemic vein pair represents a two-element unit, whose fluid mass and acceleration forces are disregarded [167]. In the context of blood losses and fluid resuscitation, HCT invariably drops such that the lessened blood viscosity is considered to have negligible effects on resistance [168]. Three segments concur to model the pulmonary circulation (i.e., pulmonary artery, capillary bed, and veins), where each segment consists in a two-element unit. The interstitial space was modeled so as to elucidate fluid shifts between the different compartments [14]. Thus, the relations between the interstitial fluid (ISF) volume and hydrostatic and oncotic pressures are duly taken into account. Actually, the latter show a certain degree of similarity to earlier relations adopted by Barnea and Sheffer [166].

The Authors' underlying assumption is that net changes in the ISF volume can occur only thanks to fluid shifts between the intravascular and interstitial spaces. In addition, capillary permeability was assumed to be constant and independent regardless of conditions of shock or variations in colloid concentrations. Bleeding entails loss of fluids, red blood cells, and colloids as well [14]. The severity of a given hemorrhage depends on relationship between arterial-end capillary hydrostatic pressures and the variations in resistance values in response to hemorrhage (so as to assure flow). The following equations express the concentration and the amount of oxygen delivered by a deciliter of blood (Eq. (18)) [14]:

(18) $$\begin{array}{c} \left[{\text{O}}_{2}\right]=\alpha \times {\text{P}}_{{\text{O}}_{2}}+\left[\text{Hb}{\text{O}}_{2}\right],\\ \left[\text{Hb}\right]=\text{HCT}\times \left[\text{H}{\text{b}}_{\text{RBC}}\right],\\ \left[\text{Hb}{\text{O}}_{2}\right]=\text{Sa}{\text{O}}_{2}\times \text{Hb}{\text{O}}_{2\text{\_}\max}\times \left[\text{Hb}\right], \end{array}$$

where *α* is the solubility coefficient of oxygen in blood, [O_2_] is the total oxygen concentration, [HbO_2_] is the concentration of oxygen bound to hemoglobin, PO_2_ is the partial oxygen pressure, SaO_2_ is the oxygen saturation of hemoglobin [Hb], [Hb_RBC_] is the hemoglobin concentration in g/deciliter of red blood cells (RBCs), the hematocrit (HCT) is the mass of hemoglobin per deciliter of blood, and HbO_2_max_ is the maximum oxygen-carrying capacity of Hb [14]. In this model, total oxygen content of blood is calculated as the sum of oxygen dissolved in the blood and oxygen transported by RBCs. In systemic arteries, hemoglobin saturation was assumed to be complete and the oxygen concentration per unit volume of RBCs was considered constant [14].

The oxygen delivery rate [*D*_*O*_2__] as a function of CO at any given time *t* is expressed as [14]:

(19) $$\begin{array}{c} D_{O_{2}}\left(t\right)=\left[O_{2}\left(t\right)\right]\times \text{CO}\left(t\right). \end{array}$$

The described model was used to study the normal hemodynamic response, the bleeding phase, bleeding control, and the monitoring phase without treatment, the fluid resuscitation phase, and the follow-up phase. Class II, III, and IV hemorrhages were simulated to study their effects on hemodynamic variables. The simulation sequences were repeated for each class of hemorrhage applying a wide range of infusion rates [14].

#### 4.4.2. Fluid Exchange

The fluid exchange model assumes the concentration of colloids in the interstitial space is constant (2%, [166]) with no leakage of colloids from the intravascular into the interstitial compartment [14]. The volumes of plasma and RBCs are calculated separately. For the plasma volume during conditions of hemorrhage, see equation (10) in Table 1, which takes into account the combined effects of fluid volume losses from bleeding and the subsequent fluid exchanges with the interstitial space [14]. In equation (10), *Q*_bleed_(*t*) is the bleeding-volume rate which comprises both plasma and red blood cell losses. Whereas RBC losses are assumed to occur only during hemorrhagic phases, HCT levels vary during hemorrhage as well as throughout fluid resuscitation [14]. See also Table 1 for calculations of red blood cell volume losses, i.e., equation (11), while blood oncotic pressure is expressed by the concentration of colloids according to equation (5). The variation in blood proteins concentration during both hemorrhage and fluid resuscitation is assumed to be proportional to the value of HCT, as computed by *C*_col_B_(*t*) = *C*_col_B_norm_ · (HCT(*t*)/HCT_norm_) (equation (12), [169]). The total weight of blood proteins is given by *W*_prot_B_(*t*) = *C*_col_B_(*t*) · *V*_plasma_(*t*) [14].

During colloid fluid infusions, the plasma colloid concentration is increased as a function of the fluid infusion rate. The weight of infused colloids is calculated as *W*_col_B_inf_(*t*) = *C*_inf_ · *V*_inf_(*t*) [14]. Similarly, the concentration of blood colloids, under conditions of controlled hemorrhage and colloid fluid treatment, is expressed as follows: *C*_col_B_(*t*) = (*W*_prot_B_(*t*) + *W*_col_B_inf_(*t*))/(*V*_plasma_(*t*)) [14]. In this expression, *V*_plasma_(*t*) was computed by the integral of equation (12) which accounts for the combined effect resulting from infusion and fluid exchanges with the interstitial compartment [14]. Fluid exchange between the intravascular and interstitial compartments is given by net filtration of fluid as blood flows along the capillary vessel (see equation (8)). The fluid moves from one compartment to another through an exchange resistance *R*_exch_ (considered constant and equal for both capillary ends) [14]. The flow of fluid at each capillary end is composed of two components: one is proportional to the hydrostatic pressure difference, and the second component is proportional to the difference in oncotic pressure [14].

### 4.5. Batzel

In their paper [12], Batzel et al. explicitly focus on modeling the behavior of the Cardiovascular System (CVS) with particular regard to hemorrhage-induced control system responses. The Authors consider a single feedback loop so as to study the impact of increased heart rate on stabilizing arterial blood pressure in response to acute hemorrhage of various degrees. A reference to future applications regards implementing additional control elements and the investigation of transfusion mechanisms in the clinical setting.

We will recapitulate the contents, in an effort to highlight those aspects that the Authors deemed most salient. In [4] Guyton illustrates *P*_*as*_ response curves to various degrees of blood loss from hemorrhage, in both compensated and uncompensated conditions. Compensatory mechanisms consist of a number of key control loops (i.e., (1) baroreceptor reflexes, (2) hormonal vasoconstrictors, (3) chemoreceptor reflexes, and (4) autotransfusion (transcapillary refill) of interstitial fluids [171]) aimed at stabilizing the CVS during bleeding.

The Authors derived the fundamental model equations and their underpinnings (see Fig. 3 in Batzel et al., [12], p. 3) by starting from the cardiovascular system and taking account the lungs (*F*_*p*_) as well as tissue compartments (*F*_*s*_) [12, 93, 172, 173]:

(20) $$\begin{array}{c} c_{\text{as}}{\dot{P}}_{\text{as}}=Q_{l}-F_{s}, \end{array}$$

(21) $$\begin{array}{c} c_{\text{vs}}{\dot{P}}_{\text{vs}}=F_{s}-Q_{r}, \end{array}$$

(22) $$\begin{array}{c} c_{\text{vp}}{\dot{P}}_{\text{vp}}=F_{p}-Q_{l}, \end{array}$$

(23) $$\begin{array}{c} c_{\text{ap}}{\dot{P}}_{\text{ap}}=F_{p}-Q_{r}, \end{array}$$

(24) $$\begin{array}{c} {\dot{S}}_{l}=\sigma_{l}, \end{array}$$

(25) $$\begin{array}{c} {\dot{S}}_{r}=\sigma_{r}, \end{array}$$

(26) $$\begin{array}{c} {\dot{\sigma }}_{l}=-\gamma_{l}\sigma_{l}-\alpha_{l}S_{l}+\beta_{l}H, \end{array}$$

(27) $$\begin{array}{c} {\dot{\sigma }}_{r}=-\gamma_{r}\sigma_{r}-\alpha_{r}S_{r}+\beta_{r}H, \end{array}$$

(28) $$\begin{array}{c} \dot{H}=u_{1}, \end{array}$$

(29) $$\begin{array}{c} {\dot{c}}_{\text{vs}}=u_{2}. \end{array}$$

The model equations are mainly due to the work of Grodins [1, 66, 143] and Kappel and Peer [80, 81]. In particular, the Authors conceptualized the cardiovascular system as a systemic and pulmonary circuit, connected in series and two hearts (left and right ventricle) that pump the blood within them.

Equations (20) and (21) represent mass balance equations for blood flowing through the arterial systemic (as) and venous systemic (vs) compartment, respectively, while equation (22) gives the mass balance equation for the venous pulmonary (vp) component.

Assuming that the volume of circulating blood is a constant, the arterial pulmonary (ap) pressure is given by equation (23).

Cardiac output can vary by modifying heart rate (*H*) or contractility (*S*). The Bowditch effect defines the relationship of proportionality between *H* and *S*. Equations (24)–(27) reflect that left (*S*_*l*_) and right (*S*_*r*_) contractilities of the ventricles are determined by the heart rate.

Table 2 succinctly defines the cardiovascular parameters adopted by Batzel et al. [12].  Table 3 lists the values of these parameters, where *c*_as_, *c*_vs_, *c*_ap_, and *c*_vp_ express the capacitances of the different compartments of the cardiovascular system.

Via Ohm's law, equations (30) and (31) define blood flow *F*, where *P*_*a*_ is arterial blood pressure, *P*_*v*_ is venous pressure, and *R*_*s*_ and *R*_*p*_ represent the systemic and pulmonary resistances, respectively. Details can be found in [12, 80, 174].

(30) $$\begin{array}{c} F_{s}=\frac{P_{\text{as}}-P_{\text{vs}}}{R_{s}}, \end{array}$$

(31) $$\begin{array}{c} F_{p}=\frac{P_{\text{ap}}-P_{\text{vp}}}{R_{p}}. \end{array}$$

Left (*Q*_*l*_) and right (*Q*_*r*_) heart cardiac outputs are defined as the mean blood flow over the length of a pulse [12]:

(32) $$\begin{array}{c} Q_{l}\left(t\right)=H\cdot V_{\text{str}\left(l\right)}=H\cdot \frac{c_{l}P_{\text{vp}}\left(t\right)f\left(S_{l}\left(t\right),P_{\text{as}}\left(t\right)\right)\left(1-k_{l}\right)}{P_{\text{as}}\left(t\right)\left(1-k_{l}\right)+f\left(S_{l}\left(t\right),P_{\text{as}}\left(t\right)\right)k_{l}},\\ Q_{r}\left(t\right)=H\cdot V_{\text{str}\left(r\right)}=H\cdot \frac{c_{r}P_{\text{vs}}\left(t\right)f\left(S_{r}\left(t\right),P_{\text{ap}}\left(t\right)\right)\left(1-k_{r}\right)}{P_{\text{ap}}\left(t\right)\left(1-k_{r}\right)+f\left(S_{r}\left(t\right),P_{\text{ap}}\left(t\right)\right)k_{r}}. \end{array}$$

*V*_str_ is the stroke volume, and it is a function of contractility *S*, intraventricular pressure *P*_*a*_ and *P*_*v*_, and time of diatole *t*_*d*_, etc. The formula *f* is a minimum function to exclude values for *V*_str_ [80] greater than filling volume. In detail, *k*_*l*_, *k*_*r*_, and *f* are defined as [12]:

(33) $$\begin{array}{c} k_{l}=\exp\left(-\frac{t_{d}}{R_{l}c_{l}}\right),\\ k_{r}=\exp\left(-\frac{t_{d}}{R_{r}c_{r}}\right),\\ f\left(s,p\right)=0.5\left(s+p\right)-0.5{\left({\left(p-s\right)}^{2}+0.01\right)}^{1/2}, \end{array}$$

Instead, for *t*_*d*_, we have the following equation [80]:

(34) $$\begin{array}{c} t_{d}=t_{c}-t_{s}, \end{array}$$

where

(35) $$\begin{array}{c} t_{c}=\frac{60}{H} \end{array}$$

is the duration of heart cycle and *t*_*s*_ is the duration of the systole. Using the empirical formula [80]:

(36) $$\begin{array}{c} t_{s}=\kappa \cdot t_{c}^{1/2}=\kappa {\left(\frac{60}{H}\right)}^{1/2}, \end{array}$$

where *κ* is a constant with 0.3 ≤ *κ* ≤ 5, we obtain [12]:

(37) $$\begin{array}{c} t_{d}=t_{d}\left(H\right)=\frac{60}{H}-\kappa {\left(\frac{60}{H}\right)}^{1/2}. \end{array}$$

Equations (28) and (29) are the control equations of the model [12]:

(38) $$\begin{array}{c} \dot{H}=u_{1},{\dot{c}}_{vs}=u_{2}, \end{array}$$

where in particular *u*_1_ and *u*_2_ represent the temporal variations in heart rate *H* and venous compliance *c*_*vs*_. The controls *u*_1_ and *u*_2_ are derived by way of the cost functional [12]:

(39) $$\begin{array}{c} \int_{0}^{\infty }q_{a}{\left(P_{\text{as}}-P_{\text{as}}^{f}\right)}^{2}+q_{v}{\left(P_{\text{vs}}-P_{\text{vs}}^{f}\right)}^{2}+q_{1}{\left(u_{1}\right)}^{2}+q_{2}{\left(u_{2}\right)}^{2}dt, \end{array}$$

which optimizes the system. Feedback control can be obtained by linearizing around a steady state and applying a Riccati algebraic equation to derive the feedback gain matrix. According to finite-dimensional control system theory, this control will be suboptimal [175].

#### 4.5.1. Modeling Hemorrhage

In modeling hemorrhage, the Authors argue that the following points must be considered [12]:

1. Site and rate of bleeding from the cardiovascular system
2. Modeling of the transcapillary refill
3. How to implement a transfusion
4. How to implement hemorrhagic shock: cardiocirculatory system deterioration, physiological function of the organs, and maximum heart rate
5. Implementation of inefficiencies in system functioning due to blood loss, filling pressure, or increased heart rate produced solely by baroreflex and/or hormonal mechanisms

In particular, the Authors argue that [12]:

1. Arterial blood loss should be modeled so that the loss rate, blood volume, and pressure decrease together
2. Even though transcapillary refill only restores about 15% of blood plasma volume, it is a crucial factor in stabilizing blood pressure and ultimately should be modeled
3. There are a number of options as to the type of fluid and regimen to be considered in a transfusion
4. A characteristic feature of hemorrhagic shock is reduced cardiac performance due to insufficient cardiac perfusion. Therefore, there can be either ischemia or dysfunction due to deviations from optimal *CO*_2_ and *O*_2_ levels
5. Once the maximum sustainable heart rate is surpassed, further reductions in blood volume will tend to imply a new steady state at a reduced *P*_*as*_
6. Thus the system may stabilize at a lower *P*_*as*_ or continue to deteriorate with ongoing volume losses and/or system performance is compromised with cardiocirculatory shock. Apart from human and animal studies, data from hypovolemia in dialysis patients can provide some human corroboration of simulated results. The Authors cite a review by Cooke et al. [176] to justify the use of lower-body negative pressure (LBNP) in order to perturb homeostasis in the cardiovascular system and study hemorrhagic shock in humans

According to Secher et al. [177], three distinct stages characterize the heart rate response to reversible hypovolemia can be identified. The first stage corresponds to a loss of up to 15% of circulating blood volume. Under these conditions, there is a slight increase of heart rate (<100 beats/min) and total peripheral resistance that can compensate for the loss of blood; arterial pressure is relatively maintained (preshock). The second stage occurs with a reduction in a blood volume of approximately 30%. Such a blood loss leads at a decrease in heart rate, total peripheral resistance, and blood pressure due to C-fibres from the left ventricle [177] (i.e., von Betzold-Jarisch reflex). During the third phase, there is a further drop in blood pressure due to protracted bleeding with increased tachycardia (>120 beats/min).

In control and hemorrhage algorithm, let us now summarize the feedback controls that are considered in the algorithm that simulates hemorrhage [12]:

1. At each time *t*, the control mechanisms tend to bring the system back to equilibrium, whereby arterial systemic pressure ${\bar{P}}_{\text{as}}$ equals pressure prior to hemorrhage, *P*_as,0_. In the steady-state calculation, there is one degree of freedom
2. Heart rate is characterized by a maximal sustainable value, *H*_*e*,max_
3. If at equilibrium ${\bar{P}}_{\text{as}}=P_{\text{as},0}$, we have that *H* > *H*_*e*,max_; then the control tries to rebalance the system by “picking” $\bar{H}=H_{e,\max}$

The control design ensures that the transition from an initial perturbation (which could also be an initial stationary state) *x*^*i*^ to the final state *x*^*f*^ occurs according to the algorithm described as follows [12]:

- The “initial” *x*^*i*^ and “final” *x*^*f*^ steady states are calculated: these states are characterized by variations of some parameters such as the variation in blood volume in the interval due to hemorrhage, transfusion volume, or transcapillary refill
- The control functions *u*_*i*_ are calculated as follows. We start by considering the linearized system around state *x*^*f*^ with initial condition *x*(0) = *x*^*i*^, with the cost functional in equation (39). Then the control functions *u*_*i*_ are determined by minimizing the cost functional subject to the linearized system. These control functions are defined by the feedback gain matrix (found by solving the algebraic matrix Riccati equation). In detail, *u*_*i*_ are defined as “feedback control functions”
- The nonlinear system (i.e., equation (20) to equation (29)) is stabilized by means of this control. The latter will be suboptimal, in the sense of Russell [109]. Throughout the bleed, since the blood volume keeps decreasing, the control response changes as well

We carry out the stepwise process of derivation of the control (previously described) over fixed time intervals: after each step, the control is recalculated to take into account the volume loss due to ongoing hemorrhage. The final state of the system *x*_*k*_ at the *k*_*th*_ as the step is used as the initial state for the simulation at the (*k* + 1) step. The control at the (*k*_th_ + 1) step is determined using the equilibrium calculated by means of the volume at the end of the *k*_th_ step [12].

Now, we report the hemorrhage algorithm as described by the Authors [12]:

“*The control  u* (*t*)*  at time  t* ≥ 0*  is calculated as follows:*

(Step 1) *Change of  V*_0_*  as a consequence of hemorrhage, infusion, and exchange processes with the interstitium (capillary refill, loss of crystalloid, or colloid substitutes from plasma into the interstitium).*
(Step 2) *Compute  *${\bar{x}}_{e,t}=col\;\left({\bar{P}}_{as},\cdots ,\bar{H}\right)$*  from  f*(*x*, *p*) = 0*  with  P*_*as*_ = *P*_*as*,0_*  and  *$p={\bar{p}}_{t}$.
(Step 3) *If  *$\bar{H}\leq H_{e,\max}$, *then accept  *${\bar{x}}_{e,t}$, *compute  X*_*t*_, *and set*

(40) $$\begin{array}{c} u\left(t\right)=-B^{T}X_{t}\left(x\left(t\right)-{\bar{x}}_{e,t}\right). \end{array}$$

(Step 4) *If  *$\bar{H}>H_{e,\max}$, *then calculate  *${\bar{x}}_{e,t}$*  with  *$\bar{H}=H_{e,\max}$*  and  *$p={\bar{p}}_{t}$. *Compute  X*_*t*_*  and set*

(41) $$\begin{array}{c} u\left(t\right)=-B^{T}X_{t}\left(x\left(t\right)-{\bar{x}}_{e,t}\right).” \end{array}$$

where [12] ${\bar{x}}_{e,t}$ represents the equilibrium reached by the system, at time *t*, due to adaptive control; ${\bar{p}}_{t}$ represents the parameter vector at time *t*; $A_{t}=\left(\partial f/\partial x\right)\left({\bar{x}}_{e,t},{\bar{p}}_{t}\right)$ is the system matrix for the linearized system around ${\bar{x}}_{e,t}$, with

(42) $$\begin{array}{c} \dot{x}\left(t\right)=f\left(x\left(t\right),{\bar{p}}_{t}\right)+Bu\left(t\right),\\ y\left(t\right)=Cx\left(t\right), \end{array}$$

*B* = col(0, ⋯, 0, 1) and *C* = (1, 0, ⋯, 0) are the vectors that model the cardiovascular system; *X*_*t*_ represents the vector which is Riccati's solution of the equation *A*_*t*_^*T*^*X* + *XA*_*t*_ − XBB^*T*^*X* + *C*^*T*^*C* = 0; and *H*_*e*,max_ maximal acceptable value of heart rate at equilibrium (~130 beats/min).

#### 4.5.2. Steady-State Calculations

In the calculation of the steady state, there is one degree of freedom. After choosing a value for either *H* or *P*_as_, the calculation of the steady state is reduced to solving one equation with one unknown variable [12]. Calculations for each case are given, since the control algorithm requires that *H* be varied to restore the system back to a normal *P*_as_ level, provided that *H* ≤ *H*_*e*,max_. For *H* > *H*_*e*,max_, the control is set to *H*_*e*,max_, and the normal level for *P*_as_ derives, according to the initial assumption [12].

The possibility of reducing all steady state relations to a single equation, which can be subjected to numerical analysis, indicates that there is a unique point of equilibrium in the range of admissible physiological values [12]. Moreover, this numerical calculation of the equilibrium point accrues appreciable results, in contrast to the application of numerical solvers to the steady state relations using multiple equations, in which a solution is not easily achievable [12].

The model devoid of autoregulation is considered in more detail, hypothesizing 2 different situations, in [12] to which the reader is referred for a more in-depth and comprehensive discussion of the topic.

### 4.6. Beard

Since the 1970s, there has been a lack of consensus as to the actual etiology of hypertension [11]. Nonetheless, as far as the role of the kidney is concerned, several Authors concur that the organ is pivotal in regulating blood pressure. The pivotal observation underlying the theory is the close relationships between arterial pressure and urine production. In fact, perturbations in pressure and/or changes in the rate of salt and volume intake elicit prompt adaptive responses in renal physiology [3].

Dominance of a renal function as a controller of arterial pressure has found support in computerized cardiovascular system models known as “Guyton-Coleman models” [3]. As yet, however, no such computerized model has provided an unequivocal and complete characterization of the chronic adaptations of renal function regards blood pressure control.

We will now try to briefly explain the various components that define the whole model proposed by Beard et al. [11]. The functions on which the mathematical architecture that simulates the behavior of the cardiovascular system is based will be illustrated as well.

#### 4.6.1. Model

*(1) Aorta/Large-Artery Mechanics*. Considering the aorta a simple elastic cylinder, the tension *ε* is computed as a function of volume *V*_*A*0_ [11]:

(43) $$\begin{array}{c} \varepsilon =\frac{d_{A}}{d_{0}}={\left(\frac{V_{A0}}{V_{0}}\right)}^{1/2}, \end{array}$$

where parameter *V*_0_ represents the unstressed volume and *d*_*A*_/*d*_0_ is the ratio between the diameter in stressed conditions and that in unstressed conditions. By definition, *ε* is equal to 1 in the unstressed state when *d*_*A*_ = *d*_0_. The assumed pressure-volume relationship at the aorta is expressed by the following [11]:

(44) $$\begin{array}{c} P_{A0}=\frac{V_{A0}-V_{sA0}}{C_{A\text{o}}}, \end{array}$$

where *C*_*A*o_ expresses acute compliance and *V*_*sA*0_(*t*) accounts for creep mechanics of aortic wall, simulated as follows [11]:

(45) $$\begin{array}{c} \tau_{cA0}\frac{dV_{sA0}}{dt}=V_{sA0}^{\infty }-V_{sA0},\\ V_{sA0}^{\infty }=\left(1-\frac{C_{Ao}}{C_{\infty }}\right)V_{A0}=\gamma_{A0}V_{A0}, \end{array}$$

where *τ*_*cA*0_ is the stress-relaxation time constant and *C*_*A*o_/*C*_∞_ is the acute to chronic ratio of effective vessel compliances. Notably, Equations (44) and (45) represent diverse albeit equivalent formulations of the standard linear model of vessel mechanics [11].

The model parameters concerning the size of the arteries come from pressure and aortic diameter measurements conducted on dogs, as described by Coleridge et al. [178]. It can be considered that the experiment carried out by Coleridge et al. can be mathematically simulated through this system of equations [11]:

(46) $$\begin{array}{c} \tau_{cA0}\frac{dV_{sA0}}{dt}=V_{sA0}^{\infty }-V_{sA0},\\ \frac{dV_{A0}}{dt}=C_{A\text{o}}\frac{dP_{A0}}{dt}+\frac{dV_{sA}}{dt},\\ \frac{d\varepsilon }{dt}=\frac{1}{2{\left(V_{A0}V_{0}\right)}^{1/2}}\frac{dV_{A0}}{dt}, \end{array}$$

where the measured aortic pressure waveform as a function of time is used for numerical approximations of *dP*_*A*0_(*t*)/*dt* in equation (46). The parameters *γ*_*Ao*_, *C*_*A*o_, *τ*_*cA*_, and *d*_0_ are taken from the data in Table 4; the value of *V*_0_ was set arbitrarily by assuming a 30 mm cylindrical vessel length [11]. For the full list of parameter values, see Table 4.

*(2) Kinetics of Baroreflex*. Changes in vessel wall strain are assumed to control baroreceptor kinetics via the rate of afferent impulses. The model presupposes an average strain value $\bar{\varepsilon }\left(t\right)$, which can vary, computed as follows [11]:

(47) $$\begin{array}{c} \tau_{s}\frac{d\bar{\varepsilon }}{dt}=\varepsilon -\bar{\varepsilon }. \end{array}$$

An adjustable parameter *τ*_*s*_ serves as a time constant. By way of the saturable relationship described below, the baroreceptor firing rate is assumed proportional to $\delta_{\varepsilon }=\max\left(\varepsilon -\bar{\varepsilon },0\right)$ [11]:

(48) $$\begin{array}{c} f_{\text{BR}}\left(t\right)=f_{0}s\left(t\right)\frac{\delta_{\varepsilon }\left(t\right)}{\delta_{\varepsilon }\left(t\right)+\delta_{0}}, \end{array}$$

where *s*(*t*) is the neurosensory input determined by that portion of afferent baroreceptors in the active/permissible state, whereas *δ* and *f*_0_ are parameters to be adjusted as needed. A saturating response is enforced by equation (48), which is a static nonlinearity [179]. Another assumption is that the activity of individual baroreceptors alternates, from active to inactive, at a rate proportional to the firing frequency, with the transition rate remaining constant [11]:

(49) $$\begin{array}{c} \frac{ds}{dt}=a\left(1-s\right)-bs\frac{\delta_{\varepsilon }}{\delta_{\varepsilon }+\delta_{0}}. \end{array}$$

Via measurements produced by step-wise changes in nonpulsatile carotid sinus pressure [180] as well as by *in vivo* ramps in pulsatile aortic pressure [178], the adjustable parameters (i.e., *τ*_*s*_, *δ*_*ε*_, *f*_0_, *a*, and *b*) are identified in the baroreflex afferent model [11].

*(3) Cardiac and Circulatory Mechanics*. Schematically, a closed-loop, lumped-parameter circuit is used to model circulation. This model disregards pulmonary circulation and instead equates the heart to the left ventricle represented by a time-varying elastance. The pressure generated within the left ventricle is described as follows [11]:

(50) $$\begin{array}{c} P_{\text{LV}}\left(dt\right)=E_{\text{LV}}\left(t\right)\cdot V_{\text{LV}}\left(t\right), \end{array}$$

in which *E*_LV_(*t*) indicates the left-ventricular elastance and *V*_LV_(*t*) represents the volume of blood occupying the ventricle. Via a smooth function that increases and decreases, respectively, during systole and diastole, elastance is simulated as follows [11]:

(51) $$\begin{array}{c} E_{\text{LV}}\left(\theta \right)=\left\{\begin{array}{c} \frac{\left(\left(0.75+\phi_{\text{SN}}\right)E_{\max}-E_{\min}\right)}{2}\left[1-\cos\left(\frac{\pi \theta }{T_{M}}\right)\right]+E_{\min},\;0\leq \theta \leq T_{M},\\ \frac{\left(\left(0.75+\phi_{\text{SN}}\right)E_{\max}-E_{\min}\right)}{2}\left[\cos\left(\frac{\pi \left(\theta -T_{M}\right)}{T_{M}}\right)+1\right]+E_{\min},\;T_{M}\leq \theta \leq T_{M}+T_{R},\\ E_{\min},\;T_{M}+T_{R}\leq \theta \leq 1, \end{array}\right. \end{array}$$

where *θ* ∈ (0, 1) is the elapsed fraction of the total cardiac contraction at any given moment. The factor (0.75+*ϕ*_SN_), multiplied by *E*_max_, accounts for the impact of sympathetic tone on cardiac contractility, where *ϕ*_SN_(*t*) ∈ (0, 1) is a variable equating to sympathetic drive. Under baseline conditions, *ϕ*_SN_ ≈ 0.25, whereas cardiac contractility increases by approximately 175% at maximum sympathetic stimulation.

The variable *θ* is simulated by [11]:

(52) $$\begin{array}{c} \frac{d\theta }{dt}=H, \end{array}$$

where *H* = *H*_0_ + *H*_1_(*ϕ*_SN_ − 0.25) is the heart rate, with *θ*(*t*) cyclically returning to 0 after reaching a value of 1. The parameters *H*_0_ and *H*_1_ are set such that the baseline heart frequency is 75 beats·min^−1^, increasing to 150 beats·min^−1^ under maximal sympathetic stimulation. The simulations of the circuit model are based on equations for the state variables *θ*(*t*), *V*_LV_(*t*), *V*_*A*0_(*t*), *V*_*A*_(*t*), *V*_*V*_(*t*), *V*_*sA*_(*t*), and *V*_*sV*_(*t*). The equations using the six variables relative to volume are as follows [11]:

(53) $$\begin{array}{c} \frac{dV_{\text{LV}}}{dt}=\max\left(0,\frac{P_{V}-P_{\text{LV}}}{R_{V}}\right)-\max\left(0,\frac{P_{\text{LV}}-P_{A0}}{R_{\text{out}}}\right),\\ \frac{dV_{A0}}{dt}=\max\left(0,\frac{P_{\text{LV}}-P_{A0}}{R_{\text{out}}}\right)-\frac{P_{A0}-P_{A}}{R_{Ao}},\\ \frac{dV_{A}}{dt}=\frac{P_{A0}-P_{A}}{R_{Ao}}-\frac{P_{A}-P_{V}}{r_{AR}R_{A}},\\ \frac{dV_{V}}{dt}=\frac{P_{A}-P_{V}}{r_{AR}R_{A}}-\max\left(0,\frac{P_{V}-P_{\text{LV}}}{R_{V}}\right)+Q_{\text{input}}-Q_{\text{urine}},\\ \frac{dV_{sA0}}{dt}=\frac{V_{sA0}^{\infty }-V_{sA0}}{\tau_{cA0}},\\ \frac{dV_{sV}}{dt}=\frac{V_{sV}^{\infty }-V_{sV}}{\tau_{cV}}, \end{array}$$

where *P*_LV_(t) is determined via equation (50). The flows *Q*_in_ (uptake/infusion rate) and *Q*_urine_ (urine production rate) are described below. The max(0, ·) terms in equation (53) account for the action of valves, underlying unidirectional flow [11]. The *R*_*A*o_ and *R*_*V*_ resistances remain constant, whereas other resistances and capacitances fluctuate in response to sympathetic tone and angiotensin II levels.

*C*_*A*_(*t*), *C*_*V*_(*t*), and *R*_*A*_(*t*) are given by the following equations [11]:

(54) $$\begin{array}{c} C_{A}\left(t\right)=\frac{C_{A0}}{\left(1+\alpha_{1}\phi_{\text{SN}}\left(t\right)\right)\left(1+\alpha_{3}\phi_{A2}\left(t\right)\right)},\\ C_{V}\left(t\right)=\frac{C_{V0}}{\left(1+\alpha_{1}\phi_{\text{SN}}\left(t\right)\right)\left(1+\alpha_{3}\phi_{A2}\left(t\right)\right)},\\ R_{A}\left(t\right)=R_{A0}\left(1+\alpha_{2}\phi_{\text{SN}}\left(t\right)\right)\left(1+\alpha_{4}\phi_{A2}\left(t\right)\right), \end{array}$$

where *C*_*A*0_, *C*_*V*0_, and *R*_*A*0_ are constants. Similarly, the constants *α*_1_, *α*_2_, *α*_3_, and *α*_4_ express the magnitude of the vasoconstrictor effects of sympathetic tone and angiotensin II levels. Instead, the plasmatic angiotensin II activity is expressed by the *ϕ*_*A*2_ variable [11]. Finally, *R*_*A*_ resistance is also subject to whole-body autoregulation, aptly incorporated into the Guyton-Coleman models [3, 181, 182].

The function *r*_AR_(*t*) ∈ (0, 1) represents the autoregulating mechanism that acts on the global arterial conductivity and it is described by the equations [11]:

(55) $$\begin{array}{c} \tau_{\text{AR}}\frac{r_{\text{AR}}}{dt}=r_{\text{AR}}^{\infty }-r_{\text{AR}},\\ r_{\text{AR}}^{\infty }=\frac{1}{2}\left(1+\tanh\left(\frac{\bar{F}-F_{0}}{F_{1}}\right)\right), \end{array}$$

where the mean cardiac output, whose average is in turn variable, is averaged by $\bar{F}\left(t\right)$, a variable defined by a first-order process [11]:

(56) $$\begin{array}{c} \tau_{F}\frac{d\bar{F}}{dt}=\frac{P_{A}-P_{V}}{r_{\text{AR}}R_{A}}-\bar{F}. \end{array}$$

The pressure values can be derived from the relationships below [11]:

(57) $$\begin{array}{c} P_{A0}=\frac{V_{A0}-V_{sA}}{C_{Ao}},\\ P_{A}=\frac{V_{A}}{C_{A}},\\ P_{V}=\frac{V_{V}-V_{sV}-V_{V01}}{C_{V}}, \end{array}$$

in which venous compliance, similar to that used for the aorta, is simulated using a linear formulation of stress relaxation. In particular, venous stress-relaxation kinetics are governed by *τ*_*cV*_(*V*_*sV*_/*dt*) = *V*_*sV*_^∞^ − *V*_*sV*_, where [11]:

(58) $$\begin{array}{c} V_{sV}^{\infty }=\left(1-\frac{C_{V}}{C_{\infty }}\right)\left(V_{V}-V_{V01}\right)=\gamma_{V}\left(V_{V}-V_{V01}\right). \end{array}$$

In equation (58), the constant *V*_*V*01_ represents an unstressed volume for the whole cardiovascular system. Altogether, this component of the model comprises a total of 23 parameters [11].

*(4) Autonomic System*. In the model, the variable *ϕ*_SN_ ∈ (0, 1) represents the whole-body sympathetic tone, in turn determined by the following baroreflex arc [11]:

(59) $$\begin{array}{c} \frac{d\phi_{\text{SN}}}{dt}=f_{\text{SN}}\left(1-\phi_{\text{SN}}\right)-f_{\text{BR}}\phi_{\text{SN}}. \end{array}$$

Thus, in the absence of any baroreflex activation, sympathetic tone remains below a value of 1. The parameter *f*_SN_ is a constant, with *ϕ*_SN_(*t*) = 0.25 at baseline. Thus, in response to abrupt and marked pressure drops, *ϕ*_SN_(*t*) increases fourfold at most [11].

*(5) Renin-Angiotensin System*. The state of the renin-angiotensin system is depicted by *ϕ*_*R*_(*t*) ∈ (0, 1) and *ϕ*_*A*2_ ∈ (0, 1), two variables which represent the activity of plasma renin and angiotensin II, in turn under the control of the combined actions of sympathetic tone and blood pressure via renin release. The plasma renin variable *ϕ*_*R*_(*t*) is determined by the following [11]:

(60) $$\begin{array}{c} \tau_{R}\frac{d\phi_{R}}{dt}=\phi_{R}^{\infty }-\phi_{R},\\ \tau_{P}\frac{d\bar{P}}{dt}=P_{A}-\bar{P},\\ \phi_{R}^{\infty }=\frac{1}{2}\left(1-\tanh\left(\frac{\bar{P}-g\phi_{SN}-P_{1}}{P_{2}}\right)\right), \end{array}$$

where *ϕ*_*R*_^∞^ decreases as the time-averaged arterial pressure value $\bar{P}$ increases. The underlying assumption is that the relationship between steady-state *ϕ*_*R*_ and pressure $\bar{P}$ varies with sympathetic tone. Given that plasma renin activity and angiotensin II levels follow a perfectly linearly relationship *in vivo* [183], the Authors characterized *ϕ*_*A*2_(*t*) as following *ϕ*_*R*_(*t*) according to [11]:

(61) $$\begin{array}{c} \tau_{A2}\frac{d\phi_{A2}}{dt}=\phi_{R}-\phi_{A2}. \end{array}$$

The five parameters (i.e., *τ*_*R*_, *τ*_*A*2_, g, *P*_1_, and *P*_2_) were identified through comparative simulations of pressure, frequency, and plasma renin activity in laboratory rabbits, under conditions of experimental hemorrhage with the parameter *τ*_*P*_ arbitrarily set at 15 seconds [11].

*(6) Pressure-Diuresis/Natriuresis Control*. As an underlying assumption, body-fluid volume regulation is characterized by a linear pressure-diuresis relationship [11]:

(62) $$\begin{array}{c} Q_{\text{urine}}=\left\{\begin{array}{c} 0,\;\bar{P}<P,\\ \min\left(k_{1}\cdot \left(\bar{P}-P\right),10\text{ ml}\cdot \text{mi}{\text{n}}^{-1}\right),\;\bar{P}\geq P, \end{array}\right. \end{array}$$

where *Q*_urine_ is the rate of urine production and *k*_1_ is the slope of the *Q*_urine_/pressure ratio. In the model, *P*_*s*_(*t*) represents the offset of the pressure-diuresis relationship. The latter is ultimately under the control of sympathetic tone and angiotensin II [11]:

(63) $$\begin{array}{c} P_{s}^{\infty }=P_{s,\min}+\frac{P_{s,\max}-P_{s,\min}}{2}\left(1+\tanh\left(\frac{\phi_{\text{SN}}+\phi_{A2}-\phi_{0}}{\phi_{1}}\right)\right),\\ \tau_{k}\frac{dP_{s}}{dt}=P_{s}^{\infty }-P_{s}. \end{array}$$

The parameters *P*_*s*,min_, *P*_*s*,max_, *ϕ*_0_, and *ϕ*_1_ are constants that describe how the acute pressure-diuresis relationship shifts following fluctuations in the tone variables *ϕ*_SN_ and *ϕ*_*A*2_ [11]. Thus, it is assumed that the impact on renal function by *ϕ*_SN_ and *ϕ*_*A*2_ is equal as well as additive. Equation (63) assumes that changes in sympathetic tone and the renin-angiotensin system, expressed as *P*_*s*_, occur with a time constant *τ*_*k*_ [11].

The time constant *τ*_*k*_ was determined experimentally by measuring urine production rates during blood infusions so as to induce acute increases in pressure and decreases in *ϕ*_SN_ and *ϕ*_*A*2_ [11]. The remaining part of the parameters is determined by comparing the results provided by the model with the experimental data obtained from the control mechanisms that regulate renal excretion of water and sodium (i.e., pressure diuresis and natriuresis), with angiotensin II infusion and with administration of an angiotensin-converting enzyme (ACE) inhibitor [11].

Values listed in Table 4 were guided by several data sets and prior computational models. The values of *E*_max_ and *E*_max_ were obtained from ventricular volumes appropriate for canines, in turn adapting Beard's model [184] so as to provide plausible human pressures at baseline conditions. Cardiac cycle timing parameters *T*_*M*_ and *T*_*R*_ were set to the same values used by Beard [184]. The baseline compliances (*C*_*A*o_, *C*_*V*0_), resistances (*R*_out_, *R*_*A*o_, *R*_*A*0_, *R*_*V*_), and *V*_*V*01_ were chosen in such a way as to be under baseline conditions in which the mean pressure is 100 mmHg, the diastolic and systolic pressures are 85 and 115 mmHg, respectively, and the ejection fraction is 0.58 [11].

### 4.7. Zenker

The implemented Zenker model [13], devoid of the pulmonary circulation block, was designed to reproduce the behavior of the cardiovascular system, taking into account baroreflex blood pressure control, as well as including the interactions between intravascular volume, myocardial contractility, and peripheral resistance [13]. It consists in the univentricular heart that acts as a pump connected to the systemic circulation with the large blood vessels represented by means of linear capacitors according to the Windkessel model.

Physiological control of blood pressure is largely maintained by the baroreflex mechanism. Thus, acute blood pressure changes trigger feedback loops that modulate heart rate and contractility, as well as peripheral resistance (Figure 6). Mathematically characterized as a simplified system of ordinary differential equations, this model is capable of simulating both normal functioning of the cardiovascular system and acute responses to fluid swings in intravascular volume, providing quantitative and qualitative analyses. The rationale and design of the Zenker cardiovascular system model are aimed at achieving an acceptable trade-off between complexity, physiological fidelity, and alignment with the empirical data [13].

Below, we will briefly illustrate the equations underlying the model so as to provide a sufficiently detailed mathematical treatment without losing sight of the overall basic framework. Our challenge is to provide a simple and intuitive, yet mathematically rigorous, representation of the essential elements.

#### 4.7.1. Systole

The linear relationship between the works of systolic ejection, i.e., stroke work (*W*_*S*_) and end-diastolic volume (*V*_*ED*_), is maintained in the model over a wide range of volumes [185]. This relation can be described by the following expression [13]:

(64) $$\begin{array}{c} W_{S}=c_{\text{PRSW}}\left(V_{\text{ED}}-V_{\text{E}{\text{D}}_{0}}\right), \end{array}$$

in which the slope factor is the preload recruitable stroke work (*c*_PRSW_). The volume whose intraventricular pressure equals 0 mmHg is referred to the volume axis intercept (*V*_ED_0__) of the curve [185]. Stroke work can be approximated to the work required to go from *V*_ED_ to *V*_ES_ (end-diastolic to end-systolic cardiac volumes) given arterial pressure *P*_*a*_, which is expressed by the following [13]:

(65) $$\begin{array}{c} W_{S}=-\int_{V_{\text{ED}}}^{V_{\text{ES}}}P\left(V\right)dV\approx V_{S}\left(P_{a}-P_{\text{ED}}\right), \end{array}$$

where *P*_ED_ represents the end-diastolic intraventricular pressure, with the stroke volume [13]:

(66) $$\begin{array}{c} V_{S}=V_{\text{ED}}-V_{\text{ES}}. \end{array}$$

Given that ventricular volume must be greater than or equal to *V*_ED_0__, we can define *V*_ES_ as a function of *V*_ED_ according to the equation below [13]:

(67) $$\begin{array}{c} {\tilde{V}}_{\text{ES}}\left(V_{\text{ED}}\right)=\left\{\begin{array}{c} \max\left(V_{\text{E}{\text{D}}_{0}},{\hat{V}}_{\text{ES}}\left(V_{\text{ED}}\right)\right),\;\text{if }P_{a}>P_{\text{ED}},\\ V_{\text{E}{\text{D}}_{0}},\;\text{otherwise}. \end{array}\right. \end{array}$$

By equating Equations (64) and (65) for *W*_*S*_ and solving for *V*_*S*_, we then substitute the resulting expression in equation (66) to obtain the following equation for ${\tilde{V}}_{\text{ES}}$ [13]:

(68) $$\begin{array}{c} {\tilde{V}}_{\text{ES}}\left(V_{\text{ED}}\right)=V_{\text{ED}}-\frac{c_{\text{PRSW}}\left(V_{\text{ED}}-V_{\text{E}{\text{D}}_{0}}\right)}{P_{a}-P_{\text{ED}}}. \end{array}$$

Note that ${\tilde{V}}_{\text{ES}}$ is a continuous function of *V*_ED_ since, if *V*_ED_ > *V*_ED_0__; the limit of ${\hat{V}}_{\text{ES}}\left(V_{\text{ED}}\right)$ as *P*_ED_ approaches *P*_*a*_ from below is smaller than *V*_ED_0__ [13].

#### 4.7.2. Diastole

For each stroke cycle, we can express end-diastolic volume as a function of end-systolic volume. Ventricular filling is considered a passive occurrence, through the linear inflow resistance *R*_valve_. Influx is therefore driven by the pressure differential between the central veins *P*_CVP_ and ventricular pressure *P*_LV_(*V*_LV_), through the ODE [13]:

(69) $$\begin{array}{c} \frac{dV_{\text{LV}}}{dt}=\frac{P_{\text{CVP}}-P_{\text{LV}}\left(V_{\text{LV}}\right)}{R_{\text{valve}}}. \end{array}$$

The dependence of ventricular pressure on ventricular volume, in equation (69), is governed by the exponential relationship characterized experimentally by [185]:

(70) $$\begin{array}{c} P_{\text{LV}}\left(V_{\text{LV}}\right)=P_{0_{\text{LV}}}\left(e^{k_{E_{\text{LV}}}\left(V_{\text{LV}}-V_{\text{E}{\text{D}}_{0}}\right)}-1\right). \end{array}$$

Assuming *P*_CVP_ to remain constant, equation (69) takes the general form [13]:

(71) $$\begin{array}{c} \frac{dV}{dt}=k_{1}e^{k_{2}V}+k_{3}, \end{array}$$

with the following constants [13]:

(72) $$\begin{array}{c} k_{1}=-\frac{P_{0_{\text{LV}}}}{R_{\text{valve}}}e^{-k_{E_{\text{LV}}}}V_{\text{E}{\text{D}}_{0}}\\ k_{2}=k_{E_{\text{LV}}},\\ k_{3}=\frac{P_{\text{CVP}}+P_{0_{\text{LV}}}}{R_{\text{valve}}}. \end{array}$$

By quadrature, it resolves to the following [13]:

(73) $$\begin{array}{c} V\left(t\right)=k_{3}\left(t+C\right)-\frac{1}{k_{2}}\ln\left(\frac{1-k_{1}e^{k_{2}k_{3}\left(t+C\right)}}{k_{3}}\right). \end{array}$$

We let *t* = 0 at the onset of diastole, while eliminating the unknown constant *C*, and then apply, as the initial condition, end systolic volume *V*_ES_ to obtain the equation below [13]:

(74) $$\begin{array}{c} V\left(t\right)=k_{3}t-\frac{1}{k_{2}}\ln\left(\frac{k_{1}}{k_{3}}\left(1-e^{k_{2}k_{3}t}\right)+e^{-k_{2}V_{\text{ES}}}\right)=-\frac{1}{k_{2}}\ln\left(\frac{k_{1}}{k_{3}}\left(e^{-k_{2}k_{3}t}-1\right)+e^{-k_{2}\left(V_{\text{ES}}+k_{3}t\right)}\right). \end{array}$$

Since it avoids floating point overflow in the exponential terms, the resulting expression is advantageous, in numerical terms. We assume a constant duration of systole *T*_Sys_, given that physiological variations in heart rate affect the duration of diastole much more than systole [186]. At a given heart rate *f*_HR_, the end-diastolic volume will therefore be [13]:

(75) $$\begin{array}{c} {\hat{V}}_{\text{ED}}=V\left(f_{\text{HR}}^{-1}-T_{\text{Sys}}\right), \end{array}$$

with *V*(*t*) as expressed in equation (74). For passive filling to occur, *P*_CVP_ must exceed intraventricular pressure at the onset of diastole. Equation (75) expresses *V*_ED_ as a function of *V*_ES_ through the *V*_ES_ dependency of equation (74). The overall expression for *V*_ED_ as a function of *V*_ES_ is therefore [13]:

(76) $$\begin{array}{c} {\tilde{V}}_{\text{ED}}\left(V_{\text{ES}}\right)=\left\{\begin{array}{c} {\hat{V}}_{\text{ED}},\;\text{if }P_{\text{CVP}}>P_{\text{LV}}\left(V_{\text{ES}}\right),\\ V_{\text{ES}},\;\text{otherwise}. \end{array}\right. \end{array}$$

${\hat{V}}_{\text{ED}}$ is a continuous function of *V*_ES_. Moreover, as *P*_LV_(*V*_ES_) approaches *P*_CVP_ from below, the limit of ${\tilde{V}}_{\text{ED}}$ is *V*_ES_.

#### 4.7.3. Coupling Systole and Diastole

Zenker et al. thus define a discrete dynamical system to describe *V*_ED_, or *V*_ES_, on a beat-to-beat basis. In particular, from the current end-diastolic volume *V*_ED_^*n*^, we can apply equation (67) to compute *V*_ES_^*n*^=${\tilde{V}}_{\text{ES}}\left(V_{\text{ED}}^{n}\right)$ as well as equation (76) to obtain ${\tilde{V}}_{\text{ED}}\left(V_{\text{ES}}^{n}\right)$. In aggregate, these yield the following [13]:

(77) $$\begin{array}{c} V_{\text{ED}}^{n+1}={\tilde{V}}_{\text{ED}}\left(V_{\text{ES}}^{n}\right)={\tilde{V}}_{\text{ED}}\left({\tilde{V}}_{\text{ES}}\left(V_{\text{ED}}^{n}\right)\right). \end{array}$$

Thereafter, *V*_ES_ and *V*_ED_ were converted to variables of state within a continuous time system. This allowed them to obtain a continuous dynamical system amenable to coupling. Thereby continuous representations of the physiologic control loops and simulation with available ODE software over lengthy time intervals were made possible. This was accomplished by aligning their rates of change to the average rates over an entire cardiac cycle, i.e., to values commensurate to those of a single iteration of the discrete time interval for the current *V*_ES_ and *V*_ED_ values. Thus, they obtained [13]:

(78) $$\begin{array}{c} \frac{dV_{\text{ES}}}{dt}=\left({\tilde{V}}_{\text{ES}}\left(V_{\text{ED}}\right)-V_{\text{ES}}\right)f_{\text{HR}},\\ \frac{dV_{\text{ED}}}{dt}=\left({\tilde{V}}_{\text{ED}}\left(V_{\text{ES}}\right)-V_{\text{ED}}\right)f_{\text{HR}}. \end{array}$$

Both the discrete system and the continuous one share identical sets of fixed points as shown in equations (77) and (78), respectively. Consequently, fixed points of the discrete system (equation (76)) are given by [13]:

(79) $$\begin{array}{c} V_{\text{ED}}={\tilde{V}}_{\text{ED}}\left({\tilde{V}}_{\text{ES}}\left(V_{\text{ED}}\right)\right), \end{array}$$

and by applying ${\tilde{V}}_{\text{ES}}$ to equation (79), we obtain [13]:

(80) $$\begin{array}{c} V_{\text{ES}}={\tilde{V}}_{\text{ES}}\left(V_{\text{ED}}\right)={\tilde{V}}_{\text{ES}}\left({\tilde{V}}_{\text{ED}}\left({\tilde{V}}_{\text{ES}}\left(V_{\text{ED}}\right)\right)\right)={\tilde{V}}_{\text{ES}}\left(V_{\text{ED}}\right), \end{array}$$

thus *dV*_ES_/*dt* = *dV*_ED_/*dt* = 0 at fixed points of the discrete system. Analogously, we can observe that the fixed points of equation (78) also satisfy equation (79) and are thus fixed points of equation (77) [13].

#### 4.7.4. The Systemic Circulation

In line with a simple Windkessel model, the systemic circulation consists of linear compliances that represent the large-vessel arteries of volume *V*_*a*_ and venous vessels of volume *V*_*v*_ with their respective pressures [13]:

(81) $$\begin{array}{c} P_{\alpha }=\frac{V_{\alpha }-V_{\alpha_{0}}}{C_{\alpha }}, \end{array}$$

in which *α* is interchangeable with *a* or *v*, whereas *V*_*α*_0__ is the corresponding unstressed volume, i.e., the nonzero volume at which the pressure in the respective compartment equals 0 mmHg. These pressures are expressed in the equation linking the arterial and venous compartments via a linear resistor. The latter, in turn, represents the total peripheral resistance (*R*_TPR_) that regulates capillary blood flow *I*_*C*_, expressed as [13]:

(82) $$\begin{array}{c} I_{C}=\frac{P_{a}-P_{v}}{R_{\text{TPR}}}. \end{array}$$

Cardiac output, that is the minute volume of venoarterial blood flow (*I*_CO_) generated by the heart, is thus the product of heart rate *f*_HR_ and the ejected volume (*V*_*S*_) per beat. By applying equation (66), it assumes the following form [13]:

(83) $$\begin{array}{c} I_{\text{CO}}=f_{\text{HR}}\left(V_{\text{ED}}-V_{\text{ES}}\right). \end{array}$$

Assuming conservation of volume at the nodes, variations in volume over time, in both arterial and venous compartments, can be described by the following differential equations [13]:

(84) $$\begin{array}{c} \frac{dV_{a}}{dt}=I_{C}-I_{\text{CO}},\\ \frac{dV_{v}}{dt}=-\frac{dV_{a}}{dt}+I_{\text{external}}. \end{array}$$

With reference to the venous compartment, *I*_external_ represents either a loss of blood or an intravenous infusion, whether blood, colloid, or crystalloid.

#### 4.7.5. Baroreflex Control of Blood Pressure

As a key regulatory mechanism of cardiovascular homeostasis, baroreflex control of blood pressure relies on the established representation. In particular, the central processing component of the baroreceptor sensory input is a combination of a sigmoidal nonlinearity (in our case a logistic function) and a linear system [187, 188]. For the sake of simplicity, we equated baroreflex activity to a single activating (sympathetic) output, as opposed to the more physiologically accurate interplay of stimulatory (sympathetic) and inhibitory (parasympathetic) outputs [13]. Since the Zenker model is geared for timescales well above the order of the single cardiac cycle, the linear part of the baroreflex feedback loop is simplified. As such, it displays first-order low-pass characteristics whose time constant is in the order of the slowest actuator response (unstressed venous volume control) [13]. Delays due to neural transmission of baroreflex signaling are neglected. Given the above data, the temporal evolution of stimulatory output from baroreflex central processing obeys the following differential equation [13]:

(85) $$\begin{array}{c} \frac{dS}{dt}=\frac{1}{\tau_{\text{Baro}}}\left(1-\frac{1}{1+e^{-k_{\text{width}}\left(P_{a}-P_{a_{\text{set}}}\right)}}-S\right). \end{array}$$

Via feedback loops, baroreceptor output *S*(*t*) affects heart rate *f*_HR_, total peripheral resistance *R*_TPR_, myocardial contractility *c*_PRSW_, and unstressed venous volume *V*_*v*0_ effectors/actuators. By these mechanisms, adjustments to blood pressure occur according to its current deviation from the set point, based on the linear transformations below [13]:

(86) $$\begin{array}{c} \alpha \left(t\right)=S\left(t\right)\left(\alpha_{\max}-\alpha_{\min}\right)+\alpha_{\min}, \end{array}$$

where *α* = *f*_HR_, *R*_TPR_, or *c*_PRSW_, and [13]

(87) $$\begin{array}{c} V_{v0}\left(t\right)=\left(1-S\left(t\right)\right)\left(V_{v0_{\max}}-V_{v0_{\min}}\right)+V_{v0_{\min}}. \end{array}$$

The form of equation (87) arises from the fact that venous capacitance vessels contract, thereby reducing their unstressed volume, in response to decreases in blood pressure.

By combining equations (78) and (81)–(87) as well as explicitly writing out the dependencies relevant to the coupling of the system, Zenker et al. obtained a system of five ODEs [13]:

(88) $$\begin{array}{c} \frac{dV_{\text{ES}}}{dt}=\left({\tilde{V}}_{\text{ES}}\left(V_{\text{ED}},V_{a},S\right)-V_{\text{ES}}\right)f_{\text{HR}}\left(S\right),\\ \frac{dV_{\text{ED}}}{dt}=\left({\tilde{V}}_{\text{ED}}\left(V_{\text{ES}},V_{v}\right)-V_{\text{ED}}\right)f_{\text{HR}}\left(S\right),\\ \frac{dV_{a}}{dt}=\frac{P_{a}\left(V_{a}\right)-P_{v}\left(V_{v},S\right)}{R_{\text{TPR}}\left(S\right)}-\left(V_{\text{ED}}-V_{\text{ES}}\right)f_{\text{HR}}\left(S\right),\\ \frac{dV_{v}}{dt}=-\frac{dV_{a}}{dt}+I_{\text{external}}\left(t\right),\\ \frac{dS}{dt}=\frac{1}{\tau_{\text{Baro}}}\left(1-\frac{1}{1+e^{-k_{\text{width}}\left(P_{a}-P_{a_{\text{set}}}\right)}}-S\right). \end{array}$$

Of note, when *I*_external_ = 0, conservation of total intravascular volume allows elimination of one state variable (either *V*_*a*_ or *V*_*v*_) thus obtaining a four-dimensional system [13]. However, we opted for the above form of the system so as to maintain direct correspondence between anatomical entities and mathematical representation, albeit sacrificing some computational efficiency. As to the coupling of equations, one should consider that the sympathetic nervous system activity *S*, which represents a central control mechanism necessary for functional homeostasis of the cardiovascular system, links all components together [13]. The cyclical nature of both cardiac activity and circulation is, instead, reflected in the coupling between the equations describing their respective functions.

#### 4.7.6. Parameter Selection

The parameters describing the ventricular pressure-volume relationship, i.e., *P*_0_LV__, *V*_ED_0__, and *k*_*E*_LV__, were estimated from experimental data for the left ventricle, as reported by [185]. The remaining parameter values and the ranges for each model variable are shown in Table 5. The latter are derived from via hemodynamic measurements in experimental animal studies (see Table 6 for the description of parameters). When no explicit source is referenced, values are based on the Authors' understanding of physiological values for the simplified system, with no pretence of rigorous accuracy [13].

## 5. Discussion

We have collected here several mathematical models that describe the physiology of the cardiovascular system such as may be of interest, in particular, to describe the compensation response to acute blood loss. Albeit a representative and far from exhaustive sample, this collection may be nevertheless useful for investigators seeking a first approach to approach cardio-circulatory modeling.

Each model has its own peculiarities and preferential applications. The choice to adopt one model rather than another is dictated by the specific needs of the user. A crucial advantage of cardiocirculatory modelling is its potential to integrate the understanding of physiology and pathophysiology in an analytical framework so as to assist clinical decision-making.

Hence, the drive to advance from methodology and model development towards experimentation in the clinical context is perceived as becoming increasingly more important for cardiocirculatory models.

Our goal in this work was to briefly review a number of indicative and successful prototype models whose clinical use appears relatively straightforward. We have also created a web-based platform (available at http://biomatlab.iasi.cnr.it/models/login.php) where we have implemented two of the models included herein: the Guyton and the Zenker models, respectively. These two implemented models provide time courses of the state variables after allowing the user to set desired values of the physiological parameters as input.

Even though the Guyton model does offer benefits for long term predictions, providing additional physiological variables, as well as neurological and hormonal control of blood pressure, it has the drawback of being more labor-intensive to implement.

Therefore, in order to maximize clinical usefulness, physiological detail may need to be pruned, so as to obtain more practical, user-friendly models, while still providing clinically relevant predictions.

In our view, Zenker's model may respond to the requirement of keeping the number of significant variables to a minimum without sacrificing clinical plausibility.

## 6. Conclusion

The purpose of this paper is therefore to provide an overview of the most relevant mathematical model of the cardiocirculatory system present in the literature, in their original formulation. The models presented are those that, for different reasons, we have considered to be particularly useful inasmuch as they reflect research relevant to our main focus on cardiovascular dynamics, the compensatory response to the hemorrhage, and certain aspects of pulmonary physiology.

The models presented describe key aspects of the physiology: each model is unique and may be considered independently of the others, but taken globally, they indicate which elements of cardiocirculatory compensation have been considered most important in a past research work.

The introduction discusses the different categories of models presented in this review: some models are simple real-time models that can be directly applied to clinical settings, whereas others are more detailed reference models that the reader can use to obtain a better understanding of the interconnection of the underlying physiological mechanisms, as well as to choose parameters for simpler models [190].

It is clear, however, that all models are tentatives. The very complex and more complete models are not always capable of offering pertinent explanations on every physiological aspect of such a complex reality as the cardiovascular system. The simplest models, on the other hand, identify the essential variables, are easier to implement and faster, but may suffer of naivete and produce unrealistic prediction under certain circumstances.

In this inquiry, we note that not all of the models that we studied are sufficiently investigated for qualitative behavior, and furthermore, their validation against experimental data is often rudimentary.

Some, even if well thought out and structured, have not been used to produce continued simulations, but were limited only to a few minutes of forecasting, representing and comparing only a few hemodynamic variables with the corresponding experimental data.

Furthermore, almost none of these models specifically deal with the balance of body fluids: we refer to the phenomenon of transcapillary refill, which is always present and which plays a particularly relevant role in the case of major bleeding. Transcapillary refill as homeostatic mechanism deserves to be fully considered in a cardiocirculatory model that takes into account the volume of state of the body.

Some models could be improved simply by considering this physiological phenomenon as well, leading to more accurate modelling, treatment regimens, and clinical prognosis.

Mathematical modeling of cardiocirculatory mechanisms is developing considerably fast. The complexity of the phenomena, the dependence of these phenomena on the subject, and the variation over time of the subject's conditions are all circumstances that make the mathematical modeling complicated and that lead to the continuous development of models that describe particular situations or aspects. The very number of current available models hints to the possibility that a satisfactory formulation has not yet been found, particularly for what concerns the representation and forecasting of the response to hemorrhage.

## Figures and Tables

**Figure 1:** One-tank Winkessel model (adapted from Fig. 1 in Westerhof N., Lankhaar J.W., and Westerhof B.E., “The Arterial Windkessel”, Med Biol Eng Comput, 2009, 47, p. 132).

**Figure 2:** Two-element Windkessel model.

**Figure 3:** Three-element Windkessel model.

**Figure 4:** Four-element Windkessel model.

**Figure 5:** The complete mechanical system (adapted from Fig. 6 in Grodins [1], p. 96).

**Figure 6:** Schematic of model of the cardiovascular system (adapted from Fig. 2 in Zenker et al. [13], p. 2074).

**Table 1:** Model equations and list of symbols (adapted from Tab. A1 in Siam et al., [14], p. 92).

Model equations	
Systolic and diastolic pressures	
*P*_syst,*x*_(*t*) = max(*E*_max,*x*_∙*E*_*N*,*c*_(*t*_*n*_)(*V*_*x*_(*t*) − *V*_*x*,0_), 0) [14]	(1)
*P*_diast,*x*_(*t*) = *D*_1,*x*_ × 10^*γ*(*D*_2,*x*_)^∙*e*^(*D*_2,*x*_ · *V*_*x*_(*t*))^ + *D*_3,*x*_ln(*D*_4,*x*_*V*_*x*_(*t*)) [14]	(2)
*P*_*x*_(*t*) = max(*P*_syst,*x*_(*t*), *P*_diast,*x*_(*t*)) [14]	(3)
Fluid exchange	
$P_{\text{is}}=\left\{\begin{array}{c} 2.5\times 10^{-3}V_{\text{is}}-37,\text{for }V_{\text{is}}<14.8L,\\ 1.0\times 10^{-4}V_{\text{is}}-1.48,\text{otherwise} \end{array}\right.$ [170]	(4)
*π* = 0.2274∙*C*_col_^2^ + 2.1755∙*C*_col_ [170]	(5)
*J*_*a*_(*t*) = (*P*_*a*_cap_(*t*) − *P*_*a*_is_(*t*))/*R*_exch_ − (*π*_*a*_cap_(*t*) − *π*_*a*_is_(*t*))/*R*_exch_ [14]	(6)
*J*_*v*_(*t*) = (*P*_*v*_cap_(*t*) − *P*_*v*_is_(*t*))/*R*_exch_-(*π*_*v*_cap_(*t*) − *π*_*v*_is_(*t*))/*R*_exch_ [14]	(7)
*J*_cap_(*t*) = *J*_*a*_(*t*) + *J*_*v*_(*t*) [14]	(8)
Bleeding	
*Q*_bleed_(*t*) = *P*_*a*_cap_(*t*)/*R*_bleed_ [14]	(9)
*dV*_plasma_(*t*)/*dt* = −*Q*_bleed_(*t*)∙(1 − HCT(*t*)) + *J*_cap_(*t*) [14]	(10)
*dV*_RBC_(*t*)/*dt* = −*Q*_bleed_(*t*)∙HCT(*t*) [14]	(11)
Controlled hemorrhage	
*dV*_plasma_(*t*)/*dt* = *Q*_inf_(*t*) + *J*_cap_(*t*) [14]	(12)
*C*_col_B_(*t*) = (*C*_col_B_norm_ · (HCT(*t*)/HCT_norm_) · *V*_plasma_(*t*) + *C*_int_ · *V*_inf_(*t*))/*V*_plasma_(*t*) [14]	(13)
List of symbols	
Symbol	Description
*P*_syst_	Systolic pressure
*P*_dias_	Diastolic pressure
*D*	Diastolic parameter
*V*	Chamber volume
*x*	Chamber index
*E*	Elastance
*π*	Oncotic pressure
*V*_is_	Interstitial fluid volume
*C*_col_	Interstitial colloid concentration
*J*_*a*_	Arterial-end fluid transfer rate
*J*_*v*_	Venous-end fluid transfer rate
*J*_cap_	Capillary fluid transfer rate
*P*_*a*_cap_	Arterial-end hydrostatic pressure
*P*_*v*_cap_	Venous-end hydrostatic pressure
*π*_*a*_cap_	Capillary arterial end oncotic pressure
*P*_is_	Interstitial pressure
*π*_*a*_is_	Interstitial arterial-end oncotic pressure
*π*_*v*_is_	Interstitial venous-end oncotic pressure
*C*_col_is_	Interstitial colloid concentration
*R*_bleed_	Bleeding resistance
*V*_plasma_	Plasma volume
*V*_RBC_	RBC volume
HCT	Hematocrit
HCT_norm_	HCT initial value
*C*_col_B_	Blood total colloid concentration
*C*_col_B_norm_	Blood protein initial concentration
*Q*_bleed_	Bleeding rate
*Q*_inf_	Infusion rate
*C*_inf_	Infused colloid concentration
*V*_inf_	Infused volume
*R*_exch_	Fluid exchange resistance

**Table 2:** Cardiovascular parameters (adapted from Tab. 1 in Batzel et al., [12], p. 24).

Symbol	Description
*α*	Coefficient of *S* in the differential equation for *σ*
*A*_pesk_	*R*_*s*_ = *A*_pesk_*C*_v,O_2__
*β*	Coefficient of *H* in the differential equation for *σ*
frac	Upper compartment fraction of basic total prone systemic volume
*c*_as_	Capacitance of the arterial part of the systemic circuit
*c*_ap_	Capacitance of the arterial part of the pulmonary circuit
*c*_vs_	Capacitance of the venous part of the systemic circuit
*c*_vp_	Capacitance of the venous part of the pulmonary circuit
*F*_*p*_	Blood flow perfusing the lung compartment
*F*_*s*_	Blood flow perfusing the tissue compartment
*H*	Heart rate
*γ*	Coefficient of *σ* in the differential equation for *σ*
*P*_as_	Mean blood pressure in arterial region of the systemic circuit
*P*_ap_	Mean blood pressure in arterial region of the pulmonary circuit
*P*_vs_	Mean blood pressure in venous region of the systemic circuit
*P*_vp_	Mean blood pressure in venous region of the pulmonary circuit
*Q*	Cardiac output
*R*_*p*_	Resistance in the peripheral region of the pulmonary circuit
*R*_*s*_	Peripheral resistance in the systemic circuit
*S*	Ventricular contractility
*c*_*l*,*r*_	Compliance of the respective relaxed ventricle
*R*_*l*,*r*_	Total viscous resistance of the respective ventricle
*σ*	Derivative of *S*
*u*	Control function
*V*_str_	Ventricular stroke volume
*V*_0_	Total blood volume
VU	Total unstressed volume
*l*, *r*	Left and right of the heart circuit, respectively

**Table 3:** Parameter values (adapted from Tab. 2 in Batzel et al. [12], p. 24).

Parameter	Value/range	Unit
*V*_0_	5.0-2.712	l
*H*_max_	100	min^−1^
*c*_as_	0.01002	l · mmHg^−1^
*c*_vs_	0.643	l · mmHg^−1^
*c*_ap_	0.03557	l · mmHg^−1^
*c*_vp_	0.1394	l · mmHg^−1^
*R*_*s*_	18.41	mmHg·min·l^−1^
*R*_*p*_	1.965	mmHg·min·l^−1^
*α*_*l*_	89.47	min^−2^
*α*_*r*_	28.46	min^−2^
*β*_*l*_	68.71	mmHg · m^−1^
*β*_*r*_	1.66	mmHg · m^−1^
*γ*_*l*_	37.33	min^−1^
*γ*_*r*_	11.88	min^−1^
*c*_*l*_	0.01289	l · min^−1^
*c*_*r*_	0.06077	l · min^−1^
*R*_*l*_	11.350	mmHg·min·l^−1^
*R*_*r*_	4.158	mmHg·min·l^−1^

**Table 4:** Model parameters (adapted from Table 1 in Beard et al. [11], p. 5).

	Description	Unit
*Aorta/large-artery mechanics*		
*V*_0_ = 0.6875	Unstressed volumes	ml
*d*_0_ = 12	Unstressed diameter	mm
*C*_*Ao*_ = 0.007	Acute compliance	ml · mmHg^−1^
*γ*_*A*0_ = 0.40	Creep parameter of aortic wall	#
*τ*_*cA*0_ = 0.12	Time constant of stress relaxation	sec
*Kinetics of baroreflex*		
*τ*_*s*_ = 251.5	Adjustable parameter of baroreflex afferent model	sec
*a* = 0.0651	Baroreceptor activation rate	sec^−1^
*b* = 0.2004	Baroreceptor deactivation rate	sec^−1^
*δ*_0_ = 0.4965	Baroreceptor saturation constant	#
*f*_0_ = 299.8	Baroreceptor gain parameter	sec^−1^
*Cardiac and circulatory mechanics*		
*E*_max_ = 8	Maximum value of elastance	mmHg·ml^−1^
*E*_min_ = 0.25	Minimum value of elastance	mmHg·ml^−1^
*T*_*M*_ = 0.3	Cardiac cycle timing parameter	#
*T*_*R*_ = 0.15	Cardiac cycle timing parameter	#
*H*_0_ = 75	Heart rate parameter	beat · min^−1^
*H*_1_ = 100	Heart rate parameter	beat · min^−1^
*R*_out_ = 1 × 10^−4^	Aortic valve resistance	mmHg min·ml^−1^
*R*_*Ao*_ = 3 × 10^−4^	Aortic resistance	mmHg min·ml^−1^
*R*_*A*0_ = 0.01234	Large-artery resistance	mmHg min·ml^−1^
*R*_*V*_ = 3.359 × 10^−4^	Downstream venous resistance	mmHg min·ml^−1^
*C*_*A*0_ = 0.8174	Large-artery compliance	ml·mmHg^−1^
*C*_*V*0_ = 329.45	Downstream venous resistance	ml·mmHg^−1^
*V*_*V*01_ = 625.1	Unstressed volume of cardiovascular system	ml
*γ*_*V*_ = 0.40	Venous creep parameter	#
*τ*_*cV*_ = 120	Venous creep time constant	sec
*α*_1_ = 0.319	Arterial and venous compliance parameter	sec
*α*_2_ = 12.77	Arterial resistance parameter	sec
*α*_3_ = 1.027	Arterial and venous compliance parameter	sec
*α*_4_ = 2.972	Arterial resistance parameter	sec
*F*_0_ = 1125	Autoregulation parameter	ml·mm^−1^
*F*_1_ = 487.2	Autoregulation parameter	ml·mm^−1^
*τ*_AR_ = 6.455	Autoregulation parameter	min
*τ*_*F*_ = 15	Autoregulation parameter	sec
*Autonomic system*		
*f*_SN_ = 2.76	Constant parameter of baroreflex arc	sec^−1^
*Renin-angiotensin system*		
*τ*_*R*_ = 12.59	Time constant for renin production	min
*τ*_*A*2_ = 1.065	Time constant for angiotensin II production	min
*τ*_*P*_ = 15	Time constant for mean pressure calculation	sec
*P*_1_ = 19.18	Steady-state renin-angiotensin system tone	mmHg
*P*_2_ = 25.0	Steady-state renin-angiotensin system tone	mmHg
*g* = 246.6	Steady-state renin-angiotensin system tone	mmHg
*Pressure-diuresis/natriuresis control*		
*k*_1_ = 0.125	Slope of acute pressure-diuresis relationship	ml·sec^−1^·mmHg^−1^
*P*_*s*,max_ = 126.4	Maximum value for variable offset in the pressure-diuresis relationship	mmHg
*P*_*s*,min_ = 9.779	Minimum value for variable offset in the pressure-diuresis relationship	mmHg
*ϕ*_0_ = 0.1928	Long-term pressure-diuresis relationship	#
*ϕ*_1_ = 0.4813	Long-term pressure-diuresis relationship	#
*τ*_*k*_ = 10	Time constant for long-term pressure diuresis	min

**Table 5:** Parameter values (adapted from Table 2 in Zenker et al. [13], p. 2085).

Parameter	Value/range
*c*_PRSW_min__, *c*_PRSW_max__	34.5-138 erg/ml≜25.9-103.8 mmHg [185]
*R*_valve_	0.0025 mmHg·s/ml [68]
*f*_HR_min__, *f*_HR_max__	2/3-3 Hz
*T*_Sys_	4/15 s [186]
*R*_TPR_min__, *R*_TPR_max__	0.5335-2.134 mmHg·s/ml [189]
*V*_*a*_0__, *V*_*v*_0_min___, *V*_*v*_0_max___	700 ml; 2,700-3,100 ml [189]
*C*_*a*_, *C*_*v*_	4 ml/mmHg, 111 ml/mmHg [189]
*P*_*a*_set__	70 mmHg
*k*_width_	0.1838 mmHg [68]
*τ*_Baro_	20 s

**Table 6:** Variables and parameters of the cardiovascular model (adapted from Tab. 1 in Zenker et al. [13], p. 2082).

Symbol	Description
*f*_HR_	Heart rate
*T*_Sys_, *T*_Dia_	Duration of systole and diastole, respectively
*W*_*s*_	Stroke work, work of heart in a cardiac cycle
*I*_CO_	Cardiac output
*V*_*s*_	Stroke volume, volume of ejected blood in a cardiac cycle
*V*_ES_, *V*_ED_	End-systolic ventricular volume; end-diastolic ventricular volume
*V*_ED_0__, *P*_0_LV__, *k*_*E*_LV__	Constants describing passive empirical ventricular pressure/volume relationship
*R*_valve_	Hydraulic resistance to ventricular filling, with valve allowing unidirectional flow
*P*_ED_	End-diastolic pressure at the end of ventricular filling
*P*_LV_, *P*_*a*_, *P*_*V*_	Left ventricular pressure; arterial pressure; venous pressure
*V*_LV_, *V*_*a*_, *V*_*v*_	Ventricular volume; arterial volume; venous volume
*V*_*a*_0__, *V*_*V*_0__	Arterial and venous unstressed volume (at 0 mmHg of wall tension pressure), respectively
*R*_TPR_	Total peripheral/systemic hydraulic vascular resistance
*I*_*C*_	Arterial to venous compartment flow through capillary vessels
*c*_PRSW_	Preload recruitable stroke work, an index of how much contractility and stroke work increase with increasing diastolic filling
*C*_*a*_, *C*_*v*_	Arterial and venous compartment compliances, respectively
*τ*_Baro_	Baroreflex response time constant
*P*_*a*_set__	Baroreflex feedback loop set point
*k*_width_	Constant describing shape and maximal slope of logistic baroreflex nonlinearity

## Data Availability

All relevant data are within the paper.
